# A Stochastic SEIRS Epidemic Model with Infection Forces and Intervention Strategies

This article has been retracted.

**DOI:** 10.1155/2022/4538045

**Published:** 2022-01-10

**Authors:** Zhang Lijuan, Wang Fuchang, Liang Hongri

**Affiliations:** Institute of Disaster Prevention, Basic Course Teaching Department, Yanjiao Sanhe 065201, Hebei, China

## Abstract

The spread of epidemics has been extensively investigated using susceptible-exposed infectious-recovered-susceptible (SEIRS) models. In this work, we propose a SEIRS pandemic model with infection forces and intervention strategies. The proposed model is characterized by a stochastic differential equation (SDE) framework with arbitrary parameter settings. Based on a Markov semigroup hypothesis, we demonstrate the effect of the proliferation number *R*_0_^*S*^ on the SDE solution. On the one hand, when *R*_0_^*S*^ < 1, the SDE has an illness-free solution set under gentle additional conditions. This implies that the epidemic can be eliminated with a likelihood of 1. On the other hand, when *R*_0_^*S*^ > 1, the SDE has an endemic stationary circulation under mild additional conditions. This prompts the stochastic regeneration of the epidemic. Also, we show that arbitrary fluctuations can reduce the infection outbreak. Hence, valuable procedures can be created to manage and control epidemics.

## 1. Introduction

Many biological and human populations have been facing the threat of viral epidemics. The spread of such epidemics typically leads to large death tolls and significant economic and healthcare costs. The Ebola outbreak in early 2014 led to the loss of thousands of lives in Africa [1–3]. Thousands of people died as victims of SARS in early 2002 [4–7]. The H7N9 [8–11] and H5N6 [12, 13] epidemics emerge every year in southern areas of China, causing excessive poultry losses.

Recently, perturbations have been incorporated into deterministic models of pandemics under reasonable conditions. Subsequent models have been proposed under stochastic assumptions. Gray et al. [14] proposed a stochastic susceptible-infectious-susceptible (SIS) model and investigated the influence of perturbations on the contact rate. Tornatore et al. [15] devised a stochastic susceptible-infectious-recovered (SIR) framework and demonstrated the presence of a limit on the reproduction incentive. A stochastic susceptible-infected-vaccinated-susceptible (SIVS) model was created by Tornatore et al. in [16]. Ji and Jiang [17] examined the characteristics of a stochastic susceptible-infected-recovered-susceptible (SIRS) model under low perturbations. Lahrouz and Omari [18] addressed the extinction conditions within a nonlinear stochastic SIRS framework. Zhao et al. [19] examined a stochastic SIS model with inoculation. For this stochastic SIS model, Lin et al. [20] demonstrated the presence of stationary dispersion. Cai et al. [21] extended the SIRS model to account for the force of infection and the stochastic nature of the problem. Stochastic differential equations (SDEs) were used for the model construction. Mummert and Otunuga [22] investigate the scalability of an approach for solving a nonlinear system of ODEs by Euler's method. The system describes susceptible-exposed-infectious-recovered-susceptible (SEIRS) epidemic disease in the prey where the predator-prey interaction is given by the Lotka–Volterra type. All parameters grouping in the above 4 groups are discretized with a fixed step in a given interval. The parallel algorithm allows to receive a large number of solutions of the system of ODEs. Using these solutions, we can select those cases of system's parameters in which the dynamics of the population is stable and the disease is controlled. Talkibing [22] has proposed a stochastic version of a SEIRS epidemiological model for infectious diseases evolving in a random environment for the propagation of infectious diseases. This random model takes into account the rates of immigration and mortality in each compartment, and the spread of these diseases follows a four-state Markov process. Mummert and Otunuga [22] adapted generalized method of moments to identify the time-dependent disease transmission rate and time-dependent noise for the stochastic susceptible- exposed- infectious- temporarily immune- susceptible disease model (SEIRS) with vital rates. The stochasticity appears in the model due to fluctuations in the time-dependent transmission rate of the disease. The method is demonstrated with the US influenza data from 2004-2005 through 2016-2017 influenza seasons. The transmission rate and noise intensity stochastically work together to generate the yearly peaks in infections. There has been much work already done on the stochastic aspects of the epidemic model. For example, Norden [23, 24] described the stochastic SIS model as a logistic population model and investigated the distribution of the extinction times both numerically and theoretically. Ref. [25] introduced environmental stochasticity into the disease transmission term in a model for AIDS and condom use with two distinct states. In a second paper, Dalal et al. [26] introduced stochasticity into a deterministic model of internal HIV viral dynamics via the same technique of parameter perturbation into the death rate of healthy cells, infected cells, and viral particles. Another way to introduce stochasticity into deterministic models is telegraph noise where the parameters switch from one set to another according to a Markov switching process. As a special period of the development of infectious diseases, the incubation period has a far-reaching impact on the spread trend of different infectious diseases, some of which are very short and some of which are very long. However, in this study the SEIR model with stochasticity is missing or rare.

In this study, the main contributions are introducing a susceptible-exposed-infectious-recovered-susceptible (SEIRS) epidemic model with infection forces and investigating how changes in conditions, hatching time, and other parameter settings affect the epidemic dynamics. In particular, we extend the SDE formulation of Cai et al. [21] and fine-tune critical structural parameters. The remainder of this study is as follows. We infer a general deterministic SEIRS model (without perturbation) and its stochastic counterpart (with an infection force) in Section 2. In Section 3, we express the primary outcomes of our model. We briefly review the Markov semigroups in Section 4, while itemized evidences of the model primary outcomes are given in Section 5. In Section 6, we show our model outcomes on two SEIR models with contamination. In Section 7, we give a short discussion and a summary of the primary outcomes.

## 2. SEIR Epidemic Representation

We consider a pandemic of the SEIR type, where we indicate the numbers of susceptible, exposed, infectious, and recovered people by *S*, *E*, *I*, and *R*, respectively. The total population N is given by *N*=*S*+*E*+*I*+*R*. The SEIR model accepts that the recovered people might lose their immunity and reemerge in the susceptible state. The SEIR model is applicable to numerous infectious epidemics such as H7N9, bacterial loose bowels, typhoid fever, measles, dengue fever, and AIDS [21, 22, 27].

An epidemic is expected to cause increased mortality. According to the SEIR model, the epidemic dynamics are governed by the following equation:

(1) $$\begin{array}{c} \left\{\begin{array}{c} \frac{\text{d}S}{\text{d}t}=\Lambda -\mu S-\frac{\beta \left(I+\alpha E\right)}{f\left(1\right)}S+\gamma R,\\ \frac{\text{d}E}{\text{d}t}=\frac{\beta \left(I+\alpha E\right)}{f\left(I\right)}S-\mu E-\eta E,\\ \frac{\text{d}I}{\text{d}t}=\eta E-\left(\mu +\nu +\delta \right)I,\\ \frac{\text{d}R}{\text{d}t}=\nu I-\left(\mu +\gamma \right)R, \end{array}\right. \end{array}$$

where Λ, *μ*, *γ*, *δ*, *ν*, and *α* are all positive real constants. Λ is the population enrollment rate, *μ* is the normal population death rate, *ν* is the rate of recovery for infected people, *γ* is the rate of recovered people who lose immunity and become susceptible again, *δ* is the epidemic transmission rate, and *α* is a coefficient for the exposed people. See [28, 29] for more details. The infection force *H*(*I*) affects the infected people and has been proposed in earlier models as a key factor in deciding the epidemic transmission. The infection force *H*(*I*) in the model incorporates the adaptation of people to epidemics. For instance, *H*(*I*) might diminish as the number of infected people rises because of the way that the population may in general lessen the contacts rate. This has been translated as the “mental” impact [3]. This effect could be enforced by necessitating that the epidemic force *H*(*I*) expands for small I, while this force diminishes for large *I*. The infection force *H*(*I*) can be expressed as *βI*/*f*(*I*), where 1/*f*(*I*) represents the reduction in the valid contact coefficient *β* due to the intervention strategy [2]. With no such strategy, *f*(*I*)=1, the incidence rate reduces to the bilinear transmission rate *βSI*. To guarantee a non-monotonic epidemic force, two assumptions are made:

(H1) *f*(0) > 0 and *f*′(1) > 0, for *I* > 0.
  (H2) There is a strictly positive *ξ* > 0 for which (*I*/*f*(*I*))′ > 0, for 0 < *I* < *ξ* and (*I*/*f*(*I*))′<0 for *I* > *ξ*.

In the study of epidemic transmission, these assumptions portray the impact of intervention systems: if 0 < *I* < *ξ*, the frequency rate increases, while for *I* > *ξ*, the rate decreases.

To fuse the impacts of ecological changes, we define the stochastic model by bringing multiplicative force terms into the development conditions of both the susceptible and exposed populations. In this work, we assume that the epidemic transmission coefficient *β* varies about some normal incentive because of the persistent ecological variations [30]. Hence, we incorporate uncertainty into the deterministic model (1) through the perturbation of the dimensionless substantial contact coefficient *β* to become *β*+*σζ*(*t*). This perturbation leads to a system of stochastic differential equations:

(2) $$\begin{array}{c} \left\{\begin{array}{c} \frac{\text{d}S}{\text{d}t}=\Lambda -\mu S-\frac{\left(\beta +\sigma \zeta \left(t\right)\right)\left(I+\alpha E\right)}{f\left(I\right)}S+\gamma R,\\ \frac{\text{d}E}{\text{d}t}=\frac{\left(\beta +\zeta \left(t\right)\right)\left(I+\alpha E\right)}{f\left(I\right)}S-\mu E-\eta E,\\ \frac{\text{d}I}{\text{d}t}=\eta E-\left(\mu +\nu +\delta \right)I,\\ \frac{\text{d}R}{\text{d}t}=\nu I-\left(\mu +\gamma \right)R, \end{array}\right. \end{array}$$

where *ζ*(*t*) is a zero-mean unit-variance Gaussian white noise: 〈*ζ*(*t*)〉=0, 〈*ζ*(*t*) · *ζ*′(*t*)〉=*δ*(*t* − *t*′), where 〈*·*〉 denotes the ensemble mean, *δ*(·) is the Dirac *δ* function, and *σ* is the ecological perturbation power. The system of stochastic differential equations can be rewritten as follows:

(3) $$\begin{array}{c} \left\{\begin{array}{c} \text{d}S_{t}=\left(\Lambda -\mu S_{t}-\frac{\beta \left(I_{t}+\alpha E_{t}\right)}{f\left(I_{t}\right)}S_{t}+\gamma R_{t}\right)\text{d}t-\frac{\sigma \left(I_{t}+\alpha E_{t}\right)S_{t}}{f\left(I_{t}\right)}\text{d}B_{t},\\ \text{d}E_{t}=\frac{\beta \left(I_{t}+\alpha E_{t}\right)}{f\left(I_{t}\right)}S_{t}-\mu E_{t}-\eta E_{t}\text{d}t+\frac{\sigma \left(I_{t}+\alpha E_{t}\right)}{f\left(I_{t}\right)}\text{d}B_{t},\\ \frac{\text{d}I_{t}}{\text{d}t}=\eta E_{t}-\left(\mu +\nu +\delta \right)I_{t},\\ \frac{\text{d}R}{\text{d}t}=\nu I_{t}-\left(\mu +\gamma \right)R_{t}, \end{array}\right. \end{array}$$

where *B*_*t*_ is the typical 1-dimensional autonomous Wiener process demarcated on the whole probability space (Ω, *F*, {*F*_*t*_}_*t*≥0_, Prob). The white noise is related to the Wiener process by d*B*_*t*_=*ζ*(*t*)dt.

## 3. Main Results

First, we address the epidemic dynamics for a deterministic model with no perturbation [31]. We can obtain the reproduction number as follows:

(4) $$\begin{array}{c} R_{0}=\frac{\beta \left[\eta +\alpha \left(\mu +\nu +\delta \right)\right]\Lambda }{\mu^{2}\eta f\left(0\right)}. \end{array}$$

The dynamics of SEIRS model is bounded by the following equation:

(5) $$\begin{array}{c} \Gamma =\left\{\left(S,E,I,R\right)\in X:0<S+E+I+\frac{R\leq \Lambda }{\mu }\right\}\subset X \end{array}$$

**Theorem 1 .**

(I) If *R*_0_ ≤ 1, the epidemic-free equilibrium *E*_0_=(Λ/*μ*, 0,0,0) of the deterministic model (1) is globally asymptotically stable.
(II) If *R*_0_ > 1, model (1) admits a unique equilibrium *E* ^*∗*^=(*S* ^*∗*^, *E* ^*∗*^, *I* ^*∗*^, *R* ^*∗*^), which is globally asymptotically stable.
  (6) $$\begin{array}{c} R^{*}=\frac{\nu }{\mu +\gamma }I^{*},E^{*}=\frac{\mu +\nu +\delta }{\eta }I^{*},S^{*}=\frac{\left(\mu +\eta \right)\left(\mu +\nu +\delta \right)f\left(I^{*}\right)}{\beta \left[\left(\eta +\alpha \left(\mu +\nu +\delta \right)\right.\right]}. \end{array}$$

**Remark 1 .**

Theorem 1 shows that the reproduction number *R*_0_ highly influences the endemic behavior of the deterministic model. Moreover, Theorem 1 (II) implies, for *R*_0_ > 1, the persistence (or endemicity) of model (1) with simple dynamics. This, however, does not hold for the stochastic model as shown by the subsequent theorem.

Secondly, we investigate the epidemic dynamics associated with stochastic models. We define the stochastic reproduction number *R*_0_^*S*^ as follows:

(7) $$\begin{array}{c} R_{\text{0}}^{S}\text{:}=R_{0}-\frac{\beta \Lambda \left[\eta +\alpha \left(v+\delta \right)\right]}{\mu^{2}\eta f\left(0\right)}-\frac{\sigma^{2}\alpha^{2}\Lambda^{2}}{2\mu^{2}\left(\mu +\eta \right)f^{2}\left(0\right)},\\ R_{0}^{S}=\frac{2\mu f\left(0\right)\alpha \Lambda \beta -\sigma^{2}\alpha^{2}\Lambda^{2}}{2\mu^{2}\left(\mu +\eta \right)f^{2}\left(0\right)}. \end{array}$$

The next theorem describes the epidemic-free extinction states and the endemic persistent states for the stochastic model (2).

**Theorem 2 .**

Let (*S*_*t*_, *E*_*t*_, *I*_*t*_, *R*_*t*_) be a solution of model (3) with arbitrary initial values (*S*_0_, *E*_0_, *I*_0_, *R*_0_) ∈ Γ. If *R*_0_^*S*^ < 0, and *σ*^2^ < *βμf*(0)/Λ, then the model solution (*S*_*t*_, *E*_*t*_, *I*_*t*_, *R*_*t*_) satisfies the following properties:

(8) $$\begin{array}{c} \underset{t⟶\infty }{\lim}\sup\frac{\log\;E_{t}}{t}\leq -c<0,a.s.\\ \underset{t⟶\infty }{\lim}\sup\frac{\log\;I_{t}}{t}\leq \min\left\{-\left(\mu +\nu +\delta \right),-c\right\}<0,a.s.\\ \underset{t⟶\infty }{\lim}\sup\frac{\log\;R_{t}}{t}\leq \min\left\{-\left(\mu +\gamma \right),-\tilde{\lambda }\right\}<0,a.s.\\ \underset{t⟶\infty }{\lim}\frac{1}{t}\int_{0}^{t}S_{s}\text{d}s=\frac{\Lambda }{\mu ,a.s.}, \end{array}$$

where *c*=(*μ*+*η*)(1 − *R*_0_^*S*^). Eventually, the epidemic disappears with a likelihood of 1.

**Remark 2 .**

Adequate conditions are given by Theorem 2 when the solutions for model (1) are epidemic-free states a.s.; that is, practically all solutions of (1) are of the form (Λ/*μ*, 0,0,0).

**Remark 3 .**

The number of infected people *I*(*t*) of the deterministic model vanishes at any point where *R*_0_ ≤ 1 (cf. Theorem 1 (I)), while the contamination is constant at any point where *R*_0_ ≥ 1 (cf. Theorem 1 (II)).

Theorem 2, The aforementioned outcomes do not affect the stochastic model. We can easily discover precedents in which *R*_0_ ≥ 1 yet *R*_0_ ≤ 1 to the extent of the epidemic episode.

## 4. Proofs of Theorems 1 and 2

### 4.1. Preliminaries

Basic definitions and remarks on the Markov semigroups and their asymptotic characteristics [32–38] are given here to facilitate the demonstration of our results.

#### 4.1.1. Markov Semigroups

Let ∑=*B*(*𝕏*) be the *σ*− algebra of the Borel subsets of *𝕏*, and let *m* be the Lebesgue measure on (*𝕏*, Σ). For the space *L*^1^=*L*^1^(*𝕏*, Σ, *m*), let *𝔻*=*𝔻*(*𝕏*, Σ, *m*) denote the subset of all density functions, i.e.,

(9) $$\begin{array}{c} D=\left\{g\in L^{1}:\text{g}\geq 0,\left\|g\right\|=1\right\}, \end{array}$$

where the norm ‖*·*‖ is defined in *L*^1^. *A* linear operator *P*: *L*′⟶*L*′ is of the Markov type if *P*(*𝔻*) ⊂ *𝔻*.

Let *k*: *𝕏* × *𝕏*⟶[0, *∞*) be a measurable function that satisfies ∫_*X*_*k*(*x*, *y*)*m*(dx)=1 for essentially all *y* ∈ *𝕏*. The operator *Pg*(*X*)=∫_*𝕏*_*k*(*x*, *y*)*g*(*y*)*m*(dy) is thus an integral Markov operator, with a kernel *k*. Let {*P*(*t*)}_*t*≥0_ be a family of the Markov-type operators that fulfills the conditions:

1. *P*(0)=*I*  *d*;
2. *P*(*t*+*s*)=*P*(t)*P*(*s*) for all *s*, *t* > 0; and
3. The function *t*⟶*P*(*t*)*g* is continuous for each g ∈ *L*′. Then, the operator family {*P*(*t*)}_*t*≥0_ is called a Markov semigroup. This semigroup is called essential if the operator *P*(*t*) is a vital Markov operator for every *t* > 0. That is, a measurable function *k* : (0, *∞*) × *𝕏* × *𝕏*⟶[0, *∞*) exists so that $P\left(t\right)g\left(X\right)=\int_{𝕏}k\left(t,x,y\right)g\left(y\right)m\left(\text{dy}\right)$ for each g ∈ *𝔻*.

Key terms follow for the asymptotic analysis of Markov semigroups. Firstly, a density *g*^*∗*^ is said to be invariant under the Markov semigroup {*P*(*t*)}_*t*≥0_ if *P*(*t*)*g*^*∗*^=*g*^*∗*^ for every *t* > 0. Secondly, the Markov semigroup {*P*(*t*)}_*t*≥0_ is asymptotically stable if an invariant density *g*^*∗*^ exists such that $\underset{t⟶\infty }{\lim}\left\|P\left(t\right)g-g*\right\|=0$ for any g ∈ *𝔻*. If a differential equation system (e.g., a SDE model) generates the semigroup, then the asymptotic stability implies the convergence of all solutions starting from any density in D to the invariant density. Thirdly, a Markov semigroup {*P*(*t*)}_*t*≥0_ is sweeping (or zero type) with respect to a set *A* ∈ Σ if, for each g ∈ *𝔻*, $\underset{t⟶\infty }{\lim}\int_{A}P\left(t\right)g\left(X\right)m\left(\text{dX}\right)=0$.

**Remark 4 .**

A Markov semigroup that is sweeping with respect to limited measure sets possesses no invariant density [32, 34]. Thus, a positive kernel vital Markov semigroup with no invariant density can be non-sweeping with respect to smaller sets. Sweeping with respect to minimal sets is not identical to sweeping with respect to limited measure sets. While a Markov semigroup could be both repetitive and sweeping, it should be noted that dissipativity does not necessarily imply sweeping.

The next lemma characterizes Markov semigroups as asymptotically stable or sweeping [38].

**Lemma 1 .**

Assume {*P*(*t*)}_*t*≥0_ is an integral Markov semigroup having a continuous kernel *k*(*t*, *x*, *y*) for *t* > 0 and that ∫_*X*_*k*(*x*, *y*)*m*(dX)=1 for all *y* ∈ *𝕏*. Assume for every density g ∈ *𝔻* that ∫_0_^*∞*^*P*(*t*)*g*(*X*)d*t* > 0. Then, this semigroup is either asymptotically stable or sweeping with respect to minimal sets.

The fact that a Markov semigroup {*P*(*t*)}_*t*≥0_ is asymptotically stable or sweeping from an adequately large family of sets (e.g., from every minimal set) is known as the Foguel alternative [33].

#### 4.1.2. Fokker–Planck Equation

For any *A* ∈ Σ, let *P*(*t*, *x*, *y*, *z*, *A*) denote the progress likelihood work for the dissemination procedure (*S*_*t*_, *I*_*t*_, *E*_*t*_), where

(10) $$\begin{array}{c} R_{t}=N-S_{\text{t}}-E_{t}-I_{t},p\left(t,x,y,z,A\right)=\text{prob}\left(S_{t},I_{t},E_{t}\right)\in A. \end{array}$$

Assume that (*S*_*t*_, *I*_*t*_, *E*_*t*_) is a solution of (3) such that the distribution (*S*_0_, *I*_0_, *E*_0_) is uniformly continuous and with density *ν*(*x*, *y*, *z*). Thus, (*S*_*t*_, *I*_*t*_, *E*_*t*_) has a density *U*(*t*, *x*, *y*, *z*) that satisfies the Fokker–Planck equation [35, 37]:

(11) $$\begin{array}{c} \frac{\partial U}{\partial t}=\frac{1}{2}\sigma^{2}\left(\frac{\partial^{2}\left(\varphi U\right)}{\partial x^{2}}-2\frac{\partial^{2}\left(\varphi U\right)}{\partial x\;\partial y}+\frac{\partial^{2}\left(\varphi U\right)}{\partial y^{2}}\right)-\frac{\partial \left(f_{1}U\right)}{\partial x}-\frac{\partial \left(f_{2}U\right)}{\partial y}-\frac{\partial \left(f_{3}U\right)}{\partial z}, \end{array}$$

where *φ*(*x*, *y*, *z*)=*x*^2^(*y*+*αz*)^2^/*f*^2^(*y*) and *f*_1_(*x*, *y*, *z*)=Λ − *μx* − *β*(*y*+*αz*)/*f*(*y*)*x*+*γ*(*N* − *x* − *y* − *z*),

(12) $$\begin{array}{c} f_{2}\left(x,y,z\right)=\eta z-\left(\mu +\nu +\delta \right)y,\\ f_{3}\left(x,y,z\right)=\frac{\beta \left(y+\alpha z\right)}{f\left(y\right)}x-\left(\mu +\eta \right)z. \end{array}$$

Define the operator *P*(*t*) by setting *P*(*t*)*ν*(*x*, *y*, *z*)=*U*(*t*, *x*, *y*, *z*) for *ν* ∈ *𝔻*. Because the operator *p*(*t*) is a contraction on *𝔻*, it may be protracted to a contraction on *L*^1^. Thus, the operator family {*P*(*t*)}_*t*≥0_ creates a Markov semigroup, whose infinitesimal generator *A* satisfies (12), i.e.,

(13) $$\begin{array}{c} ΑV=\frac{1}{2}\sigma^{2}\left(\frac{\partial^{2}\left(\varphi U\right)}{\partial x^{2}}-2\frac{\partial^{2}\left(\varphi U\right)}{\partial x\;\partial y}+\frac{\partial^{2}\left(\varphi U\right)}{\partial y^{2}}\right)-\frac{\partial \left(f_{1}U\right)}{\partial x}-\frac{\partial \left(f_{2}U\right)}{\partial y}-\frac{\partial \left(f_{3}U\right)}{\partial z}. \end{array}$$

The adjoint of *A* is given by the following equation:

(14) $$\begin{array}{c} Α*V=\frac{1}{2}\sigma^{2}\left(\frac{\partial^{2}\left(\varphi U\right)}{\partial x^{2}}-2\frac{\partial^{2}\left(\varphi U\right)}{\partial x\;\partial y}+\frac{\partial^{2}\left(\varphi U\right)}{\partial y^{2}}\right)-\frac{\partial \left(f_{1}U\right)}{\partial x}-\frac{\partial \left(f_{2}U\right)}{\partial y}-\frac{\partial \left(f_{3}U\right)}{\partial z}. \end{array}$$

### 4.2. Proofs of Theorems 1 and 2

We give here rigorous proofs for the theoretical results of Section 3 using the preliminaries.

The deterministic SEIRS model (1) has two equilibrium states: one is the epidemic-free equilibrium *E*_0_=(Λ/*μ*, 0,0,0), which can be obtained for any parameter settings, while the other state is the endemic equilibrium $\overset{-}{E}*=\left(\mathrm{S*,E*,I*,R*}\right)$, which is a positive solution of the following scheme:

(15) $$\begin{array}{c} \left\{\begin{array}{c} \Lambda -\mu s-\frac{\beta \left(I+\alpha E\right)}{f\left(I\right)}S+\gamma R=0,\\ \frac{\beta \left(I+\alpha E\right)}{f\left(I\right)}S-\left(\mu +\eta \right)E=0,\\ \eta E-\mu I-\nu I-\delta I=0,\\ \nu I-\left(\mu +\gamma \right)R=0. \end{array}\right. \end{array}$$

The endemic equilibrium terms, namely, *S*^*∗*^,  *E*^*∗*^,  *I*^*∗*^, and *R*^*∗*^, can be expressed as follows:

(16) $$\begin{array}{c} S^{*}=\frac{\mu I^{*}f\left(I^{*}\right)}{\beta \left(I^{*}+\alpha E^{*}\right)},\\ R^{*}=\frac{\nu }{\mu +\gamma },\\ E^{*}=\frac{\mu +\nu +\delta }{\eta }I^{*}, \end{array}$$

and Λ − *ημ*^2^*f*(*I*^*∗*^)/*β*[*η*+*α*(*μ*+*ν*+*δ*]+(*μγ*/*μ*+*γ* − *βμ*)*I*^*∗*^=0.

Define *F*(*I*)=Λ − *ημ*^2^*f*(*I*^*∗*^)/*β*[*η*+*α*(*μ*+*ν*+*δ*)]+(*μγ*/*μ*+*γ* − *βμ*)*I*^*∗*^. Based on the assumption (H1), the function *F*(*I*) is decreasing. Since

(17) $$\begin{array}{c} F\left(0\right)=\Lambda -\frac{\mu^{2}\eta }{\beta \left[\eta +\alpha \left(\mu +\nu +\delta \right)\right]}f\left(0\right)\\ =\frac{\mu^{2}\eta }{\beta \left[\eta +\alpha \left(\mu +\nu +\delta \right)\right]}\left[\frac{\beta \left[\eta +\alpha \left(\mu +\nu +\delta \right)\right]\Lambda }{\mu^{2}\eta f\left(0\right)}-1\right]f\left(0\right)\\ =\frac{\mu^{2}\eta }{\beta \left[\eta +\alpha \left(\mu +\nu +\delta \right)\right]}\left[R_{0}-1\right]f\left(0\right). \end{array}$$

The equation *F*(*I*)=0 possesses a unique positive solution *I∗* if *R*_0_ > 1. Therefore, a unique endemic equilibrium $\overset{-}{E}*=\left(S*,E*,I*,R*\right)$ exists for model (1).

The next lemma demonstrates that the solutions for model (1) are limited, contained in a reduced set, and continuous for all *t* > 0.

**Lemma 2 .**

Model (1) is decidedly invariant where pulls of each solution with initial conditions begin in its state space *𝕏*. Also, every direction of model (1) will in the long run remain in a reduced subset of Γ.

**Proof**

Joining all conditions in (1) and considering *N*(*t*)=*S*(*t*)+*E*(*t*)+*I*(*t*)+*R*(*t*), we have the following:

(18) $$\begin{array}{c} \Lambda -\left(\mu +\delta \right)\text{N}\leq \frac{\text{dN}}{\text{dt}}=\Lambda -\mu \text{N}-\delta I\leq \Lambda -\mu \text{N}. \end{array}$$

Hereafter, by integrating (18), we obtain the following equation:

(19) $$\begin{array}{c} \frac{\Lambda }{\mu +\delta }+\left(N\left(0\right)-\frac{\Lambda }{\mu +\delta }\right)e^{-\left(\mu +\delta \right)t}\leq N\left(t\right)\leq \frac{\Lambda }{\mu }+\left(N\left(0\right)-\frac{\Lambda }{\mu }\right)e^{-\mu t}. \end{array}$$

This concludes the proof of the lemma.

**Remark 5 .**

Lemma 2 shows in particular that the dynamics of model (1) can be studied in the restricted set Γ obtained in (7).

#### 4.2.1. Epidemic-Free Dynamics of Model (1)

Here, the global asymptotic stability of the epidemic-free equilibrium E0 is investigated. In particular, we prove Theorem 1 (I).

**Proof**

Construct the following Lyapunov function: V (S,E,I,R) =1/2(*S* − Λ/*μ*)^2^+*θ*_1_*E*+*θ*_2_*I*,

where *θ*_1_=Λ/*μ* and $\theta_{2}=\left\{\begin{array}{c} \theta_{1}/\eta \left(\mu +\eta \right)\left(1-R_{0}\right)-\varepsilon \;\text{if}\;R_{0}<1\\ 0\;\text{if}\;R_{0}=1 \end{array}\right.$ for each adequately small *ε* > 0.

Hence, the time derivative of *V* for a solution of model (1) is as follows:

(20) $$\begin{array}{c} \frac{\text{d}V}{\text{d}t}=\left(S\;-\;\frac{\Lambda }{\mu }\right)\frac{\text{d}S}{\text{d}t}+\theta_{1}\left[\frac{\beta \left(I+\alpha E\right)}{f\left(I\right)}S-\left(\mu +\eta \right)E\right]+\theta_{2}\left[\eta E-\left(\mu +v+\delta \right)I\right]\\ =-\;µ{\left(S-\frac{\Lambda }{\mu }\right)}^{2}-\left(S-\frac{\Lambda }{\mu }\right)\frac{\beta S\left(I+\alpha E\right)}{f\left(I\right)}+\gamma R\left(S-\frac{\Lambda }{\mu }\right)+\frac{\theta_{1}\beta S\left(I+\alpha E\right)}{f\left(I\right)}-\left[\theta_{1}\left(\mu +\eta \right)-\theta_{2}\eta \right]E-\theta_{2}\left(\mu +v+\delta \right)I\\ \leq -\left[\mu +\frac{\beta \left(I+\alpha E\right)}{f\left(I\right)}\right]{\left(S-\frac{\Lambda }{\mu }\right)}^{2}+\frac{\theta_{1}\Lambda \beta -\mu f\left(I\right)\left[\theta_{1}\left(\mu +\eta \right)-\theta_{2}\eta \right]}{\mu f\left(I\right)}I-\theta_{2}\left(\mu +v+\delta \right)I, \end{array}$$

where the following is applied:

(21) $$\begin{array}{c} \frac{\beta \;S\left(I-\alpha E\right)}{f\left(I\right)}=\frac{\beta \left(I-\alpha E\right)}{f\left(I\right)}\left(S-\frac{\Lambda }{\mu }\right)+\frac{\Lambda \beta \left(I-\alpha E\right)}{\mu f\left(I\right)},\gamma \left(s-\frac{\Lambda }{\mu }\right)R\leq 0. \end{array}$$

If *R*_0_ <  1, and since *f*(*I*) = *f*(0)+ *f*′(0)*I*+*o*(*I*), we get the following:

(22) $$\begin{array}{c} \theta_{1}\Lambda \beta \;-\;µ\;f\left(I\right)\left[\theta_{1}\left(\mu +\eta \right)-\theta_{2}\eta \right]\\ =\theta_{1}\left[\Lambda \beta -\;µ\;f\left(0\right)\left(\mu +\eta \right)\right]\;+\;\mu f\left(0\right)\theta_{2}\eta \\ -\;µ\left[\theta_{1}\left(µ\;+\eta \right)-\theta_{2}\eta \right]\left[\;f^{\prime }\left(0\right)I\;+\;o\left(I\right)\right]\;\\ \leq -\;\theta_{1}µ\;f\left(0\right)\left(\mu +\eta \right)\left(1-R0\right)+\mu f\left(0\right)\theta_{2}\eta -\mu f^{\prime }\left(0\right)\left[\theta_{1}\left(\mu +\eta \right)-\theta_{2}\eta \right]I. \end{array}$$

Moreover, since $\theta_{2}=\left\{\begin{array}{cc} \theta_{1}/\eta \left(\mu +\eta \right)\left(1-R_{0}\right)-\varepsilon & if\;R_{0}<1\\ 0 & if\;R_{0}=1 \end{array}\right.$,

we have the following:

(23) $$\begin{array}{c} -\theta_{1}\mu f\left(0\right)\left(\mu +\eta \right)\left(1-R_{0}\right)+\mu f\left(0\right)\theta_{2}\eta =-\mu \eta f\left(0\right)\varepsilon ,\\ \theta_{1}\left(\mu +\eta \right)-\theta_{2}\eta =R_{0}\theta_{1}\left(\mu +\eta \right)+\varepsilon \eta . \end{array}$$

Hence, dV/dt ≤ −[*μ*+*β*(*I*+*αE*)/*f*(*I*)](*S* − Λ/*μ*)^2^ − *ηf*(0)*ε*/*f*(*I*)*I* − *θ*_2_(*μ*+*v*+*δ*)*I* − *R*_0_*θ*_1_(*μ*+*η*)+*εη*/*f*(*I*)*f*′(0)*I*^2^. Note the nonnegativity of the functions *S*, *E*, *I*,  and *R*. Also, note that the relationships in the right side of the last inequality are nonpositive; i.e., dV/dt ≤ 0, if and only if dV/dt=0 Consequently, the best invariant *S*=Λ/*μ*,  *E*=0,  *I*=0,  and *R*=0 set in {(*S*, *E*, *I*, *R*) : dV/dt=0} is a singleton {*E*_0_}.

If *R*_0_=1, then

(24) $$\begin{array}{c} \frac{\text{d}V}{\text{dt}}\leq -\left[\mu +\frac{\beta \left(I\;+\alpha E\right)}{f\left(I\right)}\right]{\left(S-\frac{\Lambda }{\mu }\right)}^{2}-\frac{\theta_{1}\left(\mu +\eta \right)}{f\left(I\right)}I^{2}f^{\prime }\left(0\right). \end{array}$$

By LaSalle's invariance principle [39, 40], the solutions of model (1) tend to *M* ⊂ {(*S*, *E*, *I*, *R*)*||S*=Λ/*μ*, *E*=0, *I*=0, *R*=0}, the biggest invariant subset of model (1). From the description of model (1), *M*={*E*_0_} is a singleton set. Thus, *E*_0_ is universally asymptotically constant on the set Γ if *R*_0_ ≤ 0.

When *R*_0_ > 1, the Jacobian of model (1) at *E*_0_ is given by the following equation:

(25) $$\begin{array}{c} J\left(E_{0}\right)=\left(\begin{array}{cccc} -\mu & \frac{-\Lambda \alpha }{\mu f\left(0\right)} & \frac{-\Lambda \beta }{\mu f\left(0\right)} & \gamma \\ 0 & -\left(\mu +\eta \right)+\;\frac{\beta \alpha \Lambda }{\mu f\left(0\right)} & \;\frac{\beta \Lambda }{\mu f\left(0\right)} & 0\\ 0 & \eta & -\left(\mu +\nu +\delta \right) & 0\\ 0 & 0 & \nu & -\left(\mu +\gamma \right) \end{array}\right), \end{array}$$

with eigenvalues −*µ* < 0, −(*µ*+*v*+*δ*) <  0, −(*μ*+*γ*) <  0, and

(26) $$\begin{array}{c} \left|\begin{array}{cc} -\left(\mu +\eta \right)+\frac{\beta \alpha \Lambda }{\mu f\left(0\right)} & \frac{\beta \alpha \Lambda }{\mu f\left(0\right)}\\ \eta & -\left(\mu +\nu +\delta \right) \end{array}\right|=\left(\mu +\eta \right)\left(\mu +v+\delta \right)-R_{0}\mu \eta =\mu \eta \left[\frac{\left(\mu +\eta \right)\left(\mu +v+\delta \right)}{\mu \eta }-R_{0}\right]. \end{array}$$

Therefore, the epidemic-free equilibrium is perturbed if *R*_0_ > (*μ*+*η*)(*μ*+*v*+*δ*)/*μη* > 1. This concludes the proof.

#### 4.2.2. Endemic Dynamics of Model (1)

Here, the global asymptotic stability of the endemic equilibrium *E*^*∗*^ is addressed. In particular, Theorem 1 (II) is proved.

**Proof**

The Jacobian of (2) at *E*^*∗*^ is as follows:

(27) $$\begin{array}{c} J\left(E*\right)=\left(\begin{array}{cccc} -\mu -\frac{\beta \left(I*+\alpha E*\right)}{f\left(I*\right)} & \frac{\beta \alpha S*}{f\left(I*\right)} & \frac{\beta S*\left(I*\right)\left[1-I*\right]}{f^{2}\left(I*\right)} & \gamma \\ \frac{\beta \left(I*+\alpha E*\right)}{f\left(I*\right)} & -\left(\mu +\eta \right) & 0 & 0\\ 0 & \eta & -\mu -\nu -\delta & 0\\ 0 & 0 & \nu & -\left(\mu +\gamma \right) \end{array}\right). \end{array}$$

The characteristic polynomial of the Jacobian *J*(*E∗*) is as follows:

(28) $$\begin{array}{c} \lambda^{4}+c_{{\;}^{1}}\lambda^{3}+c_{2}\lambda^{2}+c_{3}\lambda +c_{4}=0,\\ c_{1}=4\mu +\eta +v+\delta +\gamma +\frac{\beta \left(I*+\alpha E*\right)}{f\left(I*\right)}>0,\\ c_{2}=\left(\mu +v+\delta \right)\left(\mu +\gamma \right)+\left(2\mu +v+\delta +\gamma \right)\left(\frac{\beta \left(I*+\alpha E*\right)}{f\left(I*\right)}+2µ+\eta \right)+\left(µ+\eta \right)\left(µ+\frac{\beta \left(I*+\alpha E*\right)}{f\left(I*\right)}\right)-\frac{\beta \alpha S*}{f\left(I*\right)}\frac{\beta \left(I*+\alpha E*\right)}{f\left(I*\right)}>0,\\ c_{3}=\left(\mu +v+\delta \right)\left(\mu +\gamma \right)\left(\frac{\beta \left(I*+\alpha E*\right)}{f\left(I*\right)}+2\mu +\eta \right)+\left(2\mu +v+\delta +\gamma \right)\left(\mu +\eta \right)\left(\mu +\frac{\beta \left(I*+\alpha E*\right)}{f\left(I*\right)}\right)-\frac{\beta \alpha S*}{f\left(I*\right)}\frac{\beta \left(I*+\alpha E*\right)}{f\left(I*\right)}>0,\\ c_{4}=\left(\mu +v+\delta \right)\left(\mu +\gamma \right)\left(\frac{\beta \left(I*+\alpha E*\right)}{f\left(I*\right)}+2\mu +\eta \right)+\left(\mu +v+\delta +\mu +\gamma \right)\left[\left(\mu +\frac{\beta \left(I*+\alpha E*\right)}{f\left(I*\right)}\right)-\frac{\beta \alpha S*}{f\left(I*\right)}\frac{\beta \left(I*+\alpha E*\right)}{f\left(I*\right)}\right]>0. \end{array}$$

It can be verified that *c*_1_*c*_2_ − *c*_3_ > 0, *c*_3_(*c*_1_*c*_2_ − *c*_3_) − *c*_1_^2^*c*_4_ > 0. Hence, the asymptotic stability of *E*^*∗*^ can be determined by exploiting the Routh–Hurwitz criterion.

Now, by proving that *S∗*, *E∗*, and *I∗* of model (1) are globally asymptotically stable, we will immediately prove the same type of stability for the endemic equilibrium of model (1).

### 4.3. Proof of Theorem 2

For proving Theorem 2, we first prove the existence and uniqueness of a positive global solution for model (2).

**Theorem 3 .**

For some random initial solutions (*S*_0_, *E*_0_, *I*_0_, *R*_0_) ∈ Γ, there is an nontrivial positive solution (*S*_*t*_, *E*_*t*_, *I*_*t*_, *R*_*t*_) of model (2) for *t* ≥ 0, which stays in *X* with a likelihood of 1.

**Proof**

Let (*S*_0_, *E*_0_, *I*_0_, *R*_0_) ∈ Γ. Adding up the three equations in model (2) and using *N*_*t*_=*S*_*t*_+*E*_*t*_+*R*_*t*_+*I*_*t*_, we have d*N*_*t*_=(Λ − *μN* − *δI*)d*t*.

Then, if (*S*_0_, *E*_0_, *I*_0_, *R*_0_) ∈ *X* for all 0 ≤ *t*_1_ ≤ *t* almost surely (briefly a.s.), then we get (Λ − (*μ*+*δ*)*N*_*t*1_)dt ≤ dN_*t*1_ ≤ (Λ − *μN*_*t*1_)dt *a*.*s*.

By integration, we obtain Λ/*μ*+*δ* ≤ *N*_*s*_ ≤ Λ/*μ*. Thus, *S*_*t*1_, *E*_*t*1_, *I*_*t*1_, *R*_*t*1_ ∈ (0, Λ/*μ*] for all *t*_1_ ∈ [0, *t*] a.s. Because the model coefficients for (2) fulfill the neighborhood Lipschitz condition, an extraordinary nearby solution exists on *t*_1_ ∈ [0, *τ*_*e*_], where *τ*_*e*_ is the blast time. In this manner, the unique nearby solution of model (2) is certain by Itô's equation. Now, the global nature of this solution is shown, i.e., *τ*_*e*_=*∞* a.s. Let *n*_0_ > 0 be appropriately big so that *S*_0_,  *I*_0_, and *R*_0_ lie inside the interval [1/*n*_0_, *n*_0_]. For every integer *n* > *n*_0_, the stop times are obtained:

(29) $$\begin{array}{c} \tau_{n}=\text{inf}\left\{t\in \left[0,\tau_{e}\right]:\text{min}\left\{S_{t},E_{t},I_{t},R_{t}\right\}\leq \;\frac{1}{n}or\text{ max}\left\{S_{t},E_{t},I_{t},R_{t}\;\right\}\geq \;n\right\}. \end{array}$$

Set inf *ϕ*=*∞* (*∞* represents the empty set). *τ*_*n*_ grows as *n*⟶*∞*. Let $\tau_{\infty }=\underset{n⟶\infty }{\lim}\tau_{n}$. Then, *τ*_*∞*_ ≤ *τ*_*e*_ a.s.

In the following, we demonstrate that *τ*_*∞*_=*∞*. Assume on the contrary that this is not true. Thus, there exists a steady *T* > 0 such that Prob {*τ*_*∞*_  ≤  *t*} > *ε* for any *ε* ∈ (0,1). As a result, a whole number *n*_1_ ≥ *n*_0_ exists for which

(30) $$\begin{array}{c} \text{Prob}\left\{\tau_{n}\leq T\right\}\geq \varepsilon ,n\geq n_{1}. \end{array}$$

Describe the positive *C*^2^ function *V* : *𝔻*⟶ℝ_+_+by the following equation:

(31) $$\begin{array}{c} V\left(S,E,I,R\right)=\left(S-1-\ln\;S\right)+\left(I-1-\ln\;I\right)+\left(R-1-\ln\;R\right)+\left(I-1-\ln\;I\right). \end{array}$$

If (*S*_*t*_ , *E*_*t*_ , *I*_*t*_ , *R*_*t*_ ) ∈ *𝕏*, then by the Itô formulation, we obtain the following equation:

(32) $$\begin{array}{c} \text{d}V=\left[\left(1\;-\frac{1}{S}\right)\left(\Lambda -\mu S-\frac{\beta \left(I_{t}+\alpha E_{t}\;\right)}{f\left(I_{t}\right)}S_{t}+\gamma R_{t}\right)+\frac{\sigma^{2}{\left(I_{t}\;+\alpha E_{t}\;\right)}^{2}S_{t}^{2}}{2\;f^{2}\left(It\;\right)}\right]\text{d}t\\ +\left[\left(1-\frac{1}{E}\right)\left(\frac{\beta \left(I_{t}+\alpha E_{t}\;\right)}{f\left(I_{t}\right)}S_{t}-\left(\mu +\eta \right)E\right)\right.+\frac{\sigma^{2}{\left(I_{t}+\alpha E_{t}\;\right)}^{2}S_{t}^{2}}{f^{2}\left(I_{t}\right)}\text{d}t\\ +\left(1-\frac{1}{I}\right)\left[\eta E-\left(\mu +\nu +\delta \right)I\right]\text{d}t+\left(1-\frac{1}{R}\right)\left[\nu I-\left(\mu +\gamma \right)R\right]\text{d}t-\left[\left(1-\frac{1}{S}\right)\frac{\sigma \left(I_{t}+\alpha E_{t}\right)}{f\left(I_{t}\right)}S_{t}+\left(1-\frac{1}{I}\right)\frac{\sigma \left(I_{t}+\alpha E_{t}\right)}{f\left(I_{t}\right)}S_{t}\right]\\ \text{d}B_{t}=LV\text{d}t+\frac{\sigma \left(I_{t}-S_{t}+\alpha E_{t}\right)}{f\left(I_{t}\right)}\text{d}B_{t}, \end{array}$$

where

(33) $$\begin{array}{c} LV\;=\Lambda +4\mu +\gamma +\eta +v+\delta -\mu \left(S_{t}+E_{t}+I_{t}+R_{t}\;\right)\\ +\frac{3\sigma^{2}{\left(I_{t}+\alpha E_{t}\right)}^{2}}{f^{2}\left(I_{t}\right)}S_{t}^{2}-\frac{\beta \left(I_{t}+\alpha E_{t}\;\right)}{Ef\left(I_{t}\right)}S_{t}+\frac{\beta \left(I_{t}+\alpha E_{t}\;\right)}{f\left(I_{t}\right)}+\gamma R+\frac{\gamma R}{s}-\frac{\eta }{I}E-\frac{1}{R}\nu -\frac{\Lambda }{S}-\delta I-\gamma R-\eta E\\ <\Lambda +4\mu +\gamma +\eta +\nu +\delta +\frac{3\sigma^{2}\left(\xi^{2}+\alpha^{2}+2\alpha \right)}{f^{2}\left(\xi \right)}+\frac{2\beta \left(\xi +\alpha \right)}{f\left(\xi \right)}≔K. \end{array}$$

Replacing this inequality in equation (32), we get the following equation:

(34) $$\begin{array}{c} \text{dV}\left(S_{t},E_{t},I_{t},R_{t}\right)\leq K\text{d}t+\frac{\sigma \left(I_{t}-S_{t}\right)}{f\left(I_{t}\right)}{\text{dB}}_{t}, \end{array}$$

which implies that

(35) $$\begin{array}{c} \int_{0}^{\tau_{n}\wedge T}\text{dV}\left(S_{r},E_{r},I_{r},R_{r}\right)\leq \int_{0}^{\tau_{n}\wedge T}K\text{d}t+\int_{0}^{\tau_{n}\wedge T}\frac{\sigma \left(I_{r}-S_{r}\;\right)}{f\left(I_{r}\right)}{\text{dB}}_{r}, \end{array}$$

where *τ*_*n*_Λ*T*=min{*τ*_*n*_, *T*}. Evaluating the integrals of the last inequality gives the following equation:

(36) $$\begin{array}{c} EV\left(S_{\tau_{n^{\wedge T}}},I_{\tau_{n^{\wedge T}}},E_{\tau_{n^{\wedge T}}},R_{\tau_{n^{\wedge T}}}\;\right)\leq V\left(S_{0},E_{0},I_{0},R_{0}\right)+KT. \end{array}$$

Set Ω_*n*_= {*τ*_*n*_ ≤ *T* }. From (35), we have Prob (Ω_*n*_) ≥ *ε*. For each *w* ∈ Ω_*n*_, at least one exists among *S*_*τ*_*n*__(*w*), *E*_*τ*_*n*__(*w*), *I*_*τ*_*n*__(*w*), and *R*_*τ*_*n*__(*w*) with a value of either *n* or 1/*n*. Hence,

(37) $$\begin{array}{c} V\left(S_{\tau_{n}}\left(w\right),E_{\tau_{n}}\left(w\right),I_{\tau_{n}}\left(w\right),R_{\tau_{n}}\left(w\right)\right)\geq \left(n-1-lnn\right)\wedge \left(\frac{1}{n}-1-ln\frac{1}{n}\right). \end{array}$$

Next, from (34), we have the following:

(38) $$\begin{array}{c} V\;\left(S_{0},E_{0},I_{0},R_{0}\right)\geq E\left[\chi_{\tau n}\left(w\right)\cdot V\left(S_{\tau n}\;\left(w\right),E_{\tau n}\left(w\right),I_{\tau n}\left(w\right),R_{\tau n}\left(w\right)\right)\right]+KT\geq \varepsilon \left(n-1-\ln\;n\right)\wedge \left(\frac{1}{n}-1-\ln\frac{1}{n}\right), \end{array}$$

where *χ*_Ω*n*_ is the characteristic function of Ω_*n*_. *As* *n* ⟶ *∞*, the following contradiction is obtained:

(39) $$\begin{array}{c} \infty >V\left(S_{0},E_{0},I_{0},R_{0}\right)+KT=\infty \;a.s. \end{array}$$

Therefore, *τ*_*∞*_ = *∞*, and the solution of model (2) shall not blast within a limited time with a probability of one. The proof is complete.

**Remark 6 .**

From Theorem 1, the set is an almost surely positive invariant of the SDE (2). That is, for (*S*_0_, *E*_0_, *I*_0_, *R*_0_) ∈  Γ,

(40) $$\begin{array}{c} \text{Prob}\left\{\left(St\;,Et\;,It\;,Rt\;\right)\in \Gamma \right\}=1\forall t\geq 0. \end{array}$$

#### 4.3.1. Disease Extinction in the SDE Model

Here, Theorem 2 (I) on the disease extinction in the stochastic model (3) will be proved.

**Proof**

Based on the Itô formulation,

(41) $$\begin{array}{c} dl\;nE_{t}=\varphi \left(S_{t},E_{t},I_{t},R_{t}\right)\text{d}t+\frac{\sigma \alpha S_{t}}{f\left(I_{t}\;\right)}\;dB\;t, \end{array}$$

where *φ* : *R*3+⟶*R* is given by the following equation:

(42) $$\begin{array}{c} \varphi \left(u,v\right)\;=\frac{\beta \alpha u}{f\left(\nu \right)}-\left(\mu +\eta \right)+\frac{\sigma^{2}\alpha^{2}u^{2}}{\;2f^{2}\left(v\right)}. \end{array}$$

Hence,

(43) $$\begin{array}{c} \ln\;Et=\ln\;I0\;+\int_{0}^{t}\varphi \left(S_{s},I_{s}\right)\text{d}s+\int_{0}^{t}\frac{\sigma \alpha S_{s}}{f\left(I_{s}\right)}\text{d}B_{s}. \end{array}$$

Setting *G*(*t*)≔∫_0_^*t*^*σαS*_*s*_/*f*(*I*_*s*_)*dB*_*s*_, we have the following equation:

(44) $$\begin{array}{c} \frac{{\langle G,G\rangle }_{t}}{t}≔\frac{1}{t}\int_{0}^{t}\frac{\sigma^{2}\alpha^{2}S_{s}^{2}}{f^{2}\left(I_{s}\right)}dB_{s}\leq \frac{\sigma^{2}\alpha^{2}\Lambda^{2}}{\mu^{2}f^{2}\left(0\right)}<+\infty . \end{array}$$

From the strong law of large numbers for martingales [38], we obtain $\underset{t⟶\infty }{\lim}\text{ sup }G\left(t\right)/t=0\text{ a.s.}$

Based on (9), we have the following equation:

(45) $$\begin{array}{c} \varphi \left(Ss,Is\right)\;=\frac{\beta \alpha S_{t}}{f\left(I_{t\;}\right)}-\left(\mu +\eta \right)\;+\frac{\sigma^{2}\alpha^{2}S_{s}^{2}}{2f^{2}\left(I_{s}\right)}=-\frac{\sigma^{2}\alpha^{2}}{2}{\left(\frac{S_{t}}{f\left(I_{t}\right)}-\frac{\beta }{\sigma^{2}\alpha }\right)}^{2}+\frac{\beta^{2}}{2\sigma^{2}}-\left(µ\;+\eta \right)\leq \frac{\beta^{2}}{2\sigma^{2}}-\left(µ\;+\eta \right). \end{array}$$

It then follows from (29) that

(46) $$\begin{array}{c} \ln\;E_{t}\leq \;\ln\;I_{0}\;+\int_{0}^{t}\left[\frac{\beta^{2}}{2\sigma^{2}}-\left(\mu +\eta \right)\right]\text{d}s+G\left(t\right). \end{array}$$

If we divide both sides of (46) by *t* and let *t*⟶∞, we get the following equation:

(47) $$\begin{array}{c} \underset{t⟶\infty }{\lim}\frac{\ln\;I_{t}}{t}\leq \frac{\beta^{2}}{2\sigma^{2}}-\left(µ\;+\eta \right)a.s. \end{array}$$

Now, consider the case when *σ*^2^ < *βμf*(0)/Λ. Thus,

(48) $$\begin{array}{c} \varphi \left(S_{s},I_{s}\right)\;=-\frac{\sigma^{2}\alpha^{2}}{2}{\left(\frac{S_{t}}{f\left(I_{t}\right)}-\frac{\beta }{\sigma^{2}\alpha }\right)}^{2}+\frac{\beta^{2}}{2\sigma^{2}}-\left(\mu +\eta \right)\leq -\frac{\sigma^{2}\alpha^{2}}{2}{\left(\frac{\Lambda }{\mu f\left(0\right)}-\frac{\beta }{\sigma^{2}\alpha }\right)}^{2}+\frac{\beta^{2}}{2\sigma^{2}}-\left(µ\;+\eta \right)\\ =\frac{\Lambda \alpha \beta }{\mu f\left(0\right)}-\frac{\sigma^{2}\alpha^{2}\Lambda^{2}}{2\mu^{2}f^{2}\left(0\right)}-\left(µ\;+\eta \right)\\ =\left(µ\;+\eta \right)\left(\frac{2\mu f\left(0\right)\alpha \Lambda \beta -\sigma^{2}\alpha^{2}\Lambda^{2}}{2\mu^{2}\left(µ\;+\eta \right)f^{2}\left(0\right)}-1\right)\\ =\left(µ\;+\eta \right)\left(R_{0}^{s}-1\right), \end{array}$$

where

(49) $$\begin{array}{c} R_{0}^{s}=\frac{2\mu f\left(0\right)\alpha \Lambda \beta -\sigma^{2}\alpha^{2}\Lambda^{2}}{2\mu^{2}\left(µ\;+\eta \right)f^{2}\left(0\right)}. \end{array}$$

It then follows from (49) that

(50) $$\begin{array}{c} \ln\;I_{t}\leq \;\ln\;I_{0}+\left(\mu +\eta \right)\left(R_{0}^{s}-1\right)t\;+G\left(t\right). \end{array}$$

Therefore, from the last inequality and (10),

(51) $$\begin{array}{c} \underset{t⟶\infty }{\lim}\text{sup}\frac{\ln\;E_{t}}{t}\leq \left(µ\;+\eta \right)\left(Rs0-1\right)<0\;a.s. \end{array}$$

The reason is that *R*_0_ < 1, *R*_0_^*s*^=2*μf*(0)*α*Λ*β* − *σ*^2^*α*^2^Λ^2^/2*μ*^2^(*µ* +*η*)*f*^2^(0) < *μf*(0)*α*Λ*β*/*μ*^2^*ηf*(0)=*μα*Λ*β*/*μ*^2^*ηf*(0) < 1, and there exists a null set *N*_1_ for which Prob (*N*_1_)=0 and for any *ω* ∉ *N*_1_,

(52) $$\begin{array}{c} \underset{t⟶\infty }{\lim}\text{sup}\frac{E_{t}\left(\omega \right)}{t}<-c. \end{array}$$

Thus, for each adequately small *ε*  >  0, there is *T*_1_= *T*_1_(*ω*) for which

(53) $$\begin{array}{c} E_{t}\left(\omega \right)\leq e^{\left(-c+\varepsilon \right)t},\;\forall t\geq T1. \end{array}$$

From the 3rd equation of the stochastic model (3), for each *ω* ∈ Ω, if *t* ≥ *T*_1_(*ω*),

(54) $$\begin{array}{c} \text{It}\left(\omega \right)=e-\left(\mu +v+\delta \right)t\left(\int_{0}^{t}e^{\left(µ+v+\delta \;\right)}{\;}^{s}I_{s}\text{d}s+I_{0}\right)\\ \leq I_{0}e^{-\left(\mu +v+\delta \right)t}+\eta e^{-\left(\mu +v+\delta \right)t}\int_{0}^{t}e^{\left(µ+v+\delta \;\right)}{\;}^{s}I_{s}\text{d}s+\nu e^{-\left(\mu +v+\delta \right)t}\int_{T_{1}}^{t}e^{\left(\mu +v+\delta -c+\varepsilon \;\right)}{\;}^{s}\text{d}s. \end{array}$$

Thus, for any

(55) $$\begin{array}{c} \omega \notin N_{1},\lim\text{sup}\frac{1}{t}\ln\;I_{t}\left(\omega \right)\leq \text{min}\left\{-\left(\mu +v+\delta \right),-c+\varepsilon \right\}a.s. \end{array}$$

Letting *ε*⟶0, we get limsup(1/*t*)ln  *I*_*t*_(*ω*) ≤ min{−(*μ*+*v*+*δ*), −*c*}, *a*.*s*. Correspondingly, there is a null set *N*_2_ such that Prob (*N*_2_)=0 and for each *ω* ∉ *N*_2_,

(56) $$\begin{array}{c} \lim\sup\frac{I_{t}\left(\omega \right)}{t}<-\tilde{\lambda }\;a.s. \end{array}$$

for a constant $\tilde{\lambda }>0$. Therefore, for each adequately small *ε* > 0, there is *T*_2_=*T*_2_(*ω*) such that $I_{t}\left(\omega \right)\;\leq \;e^{\left(-\tilde{\lambda }\;+\varepsilon \right)t},\forall t\geq T_{2}.$ Similarly, we have the following equation:

(57) $$\begin{array}{c} Rt\left(\omega \right)=e-\left(\mu +\gamma \right)t\left(v\int_{0}^{t}e^{\left(µ+\gamma \;\right)}{\;}^{s}I_{s}\text{d}s+R_{0}\right)\leq R_{0}e^{-\left(µ+\gamma \right)t}\\ +ve^{-\left(\mu +\gamma \right)t}\int_{0}^{T_{2}}e^{\left(µ+\gamma \right)t}I_{s}\text{d}s+ve^{-\left(µ+\gamma \right)t}\int_{T_{2}}^{t}e^{\left(µ+\gamma -\tilde{\lambda +\varepsilon }\right)s}I_{s}\text{d}s. \end{array}$$

It follows that for any *ω* ∉ *N*_2_,

(58) $$\begin{array}{c} \lim\sup\frac{1}{t}\ln\;R_{t}\left(\omega \right)\leq \min\left\{-\left(\mu +\gamma \right),-\tilde{\lambda }+\varepsilon \right\}\;a.s. \end{array}$$

Letting *ε*⟶0, we get $lin\sup1/t\ln\;R_{t}\left(\omega \right)\leq \min\left\{-\left(\mu +\gamma \right),-\tilde{\lambda }\right\},\;a.s.$ Likewise, a null set *N*_3_ exists so that Prob (*N*_3_) = 0 and for all *ω* ∉  *N*_3_,

(59) $$\begin{array}{c} \text{lin}\sup\frac{R_{t}\left(\omega \right)}{t}<-\tilde{\lambda },\;a.s., \end{array}$$

for some constant $-\tilde{\lambda }>0.$ Thus, for any adequately small *ε*  >  0, there exists *T*_3_= *T*_3_(*ω*) for which $R_{t}\left(\omega \right)\leq e^{\left(-\tilde{\lambda }+\varepsilon \right)t}\;,\forall_{t}\geq T_{3}$. Finally, we consider *S*_*t*_. In view of the above analysis, there exists the null set *N* = *N*_1_ ∪ *N*_2_ ∪ *N*_3_ and *T*=*T* (*ω*)=max{*T*_1_, *T*_2_, *T*_3_} for which

Prob(*N*)=0 and for all *ω* ∉  *N*,

(60) $$\begin{array}{c} d\left(S_{t}+E_{t}+\;I_{t}+R_{t}\right)=\left[\Lambda -\delta I_{t}-\mu \left(S_{t}+E_{t}+\;I_{t}+R_{t}\;\right)\right]\text{d}t\geq \left(\Lambda -\delta e^{\left(-\tilde{\lambda }+\varepsilon \right)t}-\mu \left(S_{t}+E_{t}+\;I_{t}+R_{t}\;\right)\text{d}t\right.,\;\forall_{t}\geq T. \end{array}$$

This implies

(61) $$\begin{array}{c} \frac{1}{t}\int_{0}^{t}\left(S_{t}+E_{t}+\;I_{t}+R_{t}\;\right)\text{d}s\geq \frac{\Lambda }{\mu }-\frac{\delta }{t}\int_{0}^{t}e^{\left(-\tilde{\lambda }+\varepsilon \right)t}\text{d}s-\varphi \left(t\right), \end{array}$$

where

(62) $$\begin{array}{c} \varphi \left(t\right)=\frac{1}{\mu }\left(\frac{S_{t}+E_{t}+\;I_{t}+R_{t}}{t}-\frac{S_{0}+E_{0}+\;I_{0}+R_{0}}{t}\right)\text{ and }\underset{t⟶\infty }{\lim}\varphi \left(t\right)=0a.s. \end{array}$$

For a random *ε*, we have the following equation:

(63) $$\begin{array}{c} \underset{t⟶\infty }{\lim}\inf\frac{1}{t}\int_{0}^{t}\left(S_{\text{s}}+\;I_{s}+E_{s}+R_{s}\right)\text{d}s\geq \frac{\Lambda }{\mu }a.s. \end{array}$$

From Remark 6, we deduce that

(64) $$\begin{array}{c} \underset{t⟶\infty }{\lim}\frac{1}{t}\int_{0}^{t}\left(S_{\text{s}}+I_{s}+E_{s}+\;R_{s}\right)\text{d}s=\frac{\Lambda }{\mu }\;a.s. \end{array}$$

Together with the aforementioned results, we get $\underset{t⟶\infty }{\lim}\left(1/t\right)S_{s}\text{d}s=\Lambda /\mu a.s.$ Hence, the proof is finished.

#### 4.3.2. Stochastic Asymptotic Stability

In this subsection, we show that under mild additional conditions the solutions of model (2) converge to the endemic state a.s., and in particular, we prove Theorem 2 (II). We will initially demonstrate the asymptotic stability of the Markov semigroup by showing the existence of an invariant density for the semigroup.

**Lemma 3 .**

For each point (*x*_0_, *y*_0_, *z*_0_) ∈ *X* and *t* > 0, the progress likelihood work *P*(*t*, *x*_0_, *y*_0_, *z*_0_, *A*) possesses a continuous density *k*(*t*, *x*, *y*, *z*; *x*_0_, *y*_0_, *z*_0_).

**Proof**

For proving this lemma, we utilize the Hörmander hypothesis [41] on the presence of smooth densities of the change likelihood work for dispersion processes.

Let

(65) $$\begin{array}{c} a_{0}\left(S,E,I\right)\;=\left[\begin{array}{c} \Lambda -µS-\frac{\beta \;\left(I+\alpha E\right)}{f\left(I\right)}S+\gamma R\\ \frac{\beta \;\left(I+\alpha E\right)}{f\left(I\right)}S-\mu E-\eta E\\ µE-\left(\mu v+\delta \right)I \end{array}\right], \end{array}$$

and

(66) $$\begin{array}{c} a_{1}\left(S,E,I\right)\;=\left[\begin{array}{c} -\frac{\sigma \left(I+\alpha E\right)}{f\left(I\right)}S\\ \frac{\sigma \left(I+\alpha E\right)}{f\left(I\right)}S\\ 0 \end{array}\right]. \end{array}$$

By straight computations, the Lie bracket [*a*_0_, *a*_1_] is a vector field expressible as follows:

(67) $$\begin{array}{c} a_{1}=\left[a_{0},a_{1}\right]=\left[\begin{array}{c} -\sigma \frac{A_{11}}{f^{2}\left(I\right)}\\ \sigma \frac{A_{11}}{f^{2}\left(I\right)}\\ \frac{-S\left(I+\alpha E\right)\eta \sigma }{f\left(I\right)} \end{array}\right], \end{array}$$

where

(68) $$\begin{array}{c} A_{11}=\left[-\left(I^{2}\gamma +E\left(E\alpha \gamma -N\alpha \gamma +S\alpha \gamma -S\eta +S\alpha \eta -\alpha \Lambda +\;S\alpha \mu \right)\right)+I\left(\left(E-N+E\alpha \right)\gamma -\Lambda +S\left(\gamma +\delta +\mu \right)\right)\right]\;f\left(I\right)+\\ S\left(I+\alpha E\right)\left(-E\eta +I\left(v+\delta +\omega \right)\right)\;f^{\prime }\left(I\right). \end{array}$$

Set *a*_3_=[*a*_1_, *a*_2_]. The vector fields *a*_1_, *a*_2_, *a*_3_ are linearly independent on the space *X*. Hence, for all (*S*, *E*, *I*) ∈ *X*, *a*_1_, *a*_2_,  and *a*_3_ span the space *X*. Based on the Hörmander theorem [42, 43], the transition probability function *P*(*t*, *x*_0_, *y*_0_, *z*_0_, *A*) has a continuous density *k*(*t*, *x*, *y*, *z*; *x*_0_, *y*_0_, *z*_0_) and *k* ∈ *C*^*∞*^((0, *∞*) × *X* × *X*. Next, the positivity of *k* is examined using sustenance theorems [41, 44].

Pick a fixed point (*x*_0_, *y*_0_, *z*_0_) ∈ *X* and a function *φ* ∈ *L*^2^([0, *T* ], *ℝ*). Note this system of integral equations:

(69) $$\begin{array}{c} \left\{\begin{array}{c} x_{\phi }\left(t\right)=x_{0}+\int_{0}^{t}\left(f_{1}\left(x_{\phi }\left(s\right),y_{\phi }\left(s\right),z_{\phi }\left(s\right)\right)\right)-\sigma \phi \frac{x_{\phi }\left(s\right)+\alpha y_{\phi }\left(s\right)}{f\left(y_{\phi }\left(s\right)\right)}x_{\phi }\left(s\right)\text{d}s,\\ y_{\phi }\left(t\right)=y_{0}+\int_{0}^{t}\left(f_{2}\left(x_{\phi }\left(s\right),y_{\phi }\left(s\right),z_{\phi }\left(s\right)\right)\right)\sigma \phi \frac{x_{\phi }\left(s\right)+\alpha y_{\phi }\left(s\right)}{f\left(y_{\phi }\left(s\right)\right)}x_{\phi }\left(s\right)\text{d}s,\\ z_{\phi }\left(t\right)=z_{0}+\int_{0}^{t}\left(f_{3}\left(x_{\phi }\left(s\right),y_{\phi }\left(s\right),z_{\phi }\left(s\right)\right)\right)\text{d}s, \end{array}\right. \end{array}$$

where *f*_1_(*x*, *y*, *z*),  *f*_2_(*x*, *y*, *z*), and *f*_3_(*x*, *y*, *z*) are given in (11).

Let *X*=(*x*, *y*, *z*)^*T*^and *X*_0_=(*x*_0_, *y*_0_, *z*_0_)^*T*^. Let *DX*_0;*ϕ*_ be the Fréchet derivative of the *h*⟶*X*_*ϕ*_+*h*(*T*) function from *L*^2^([0, *T* ]; *ℝ*) to **X**. If for some *ϕ* ∈ *L*^2^([0, *T* ]; *ℝ*) the derivative *DX*_0;*ϕ*_ has a rank of 3, then *k*(*T*, *x*, *y*, *z*; *x*_0_, *y*_0_, *z*_0_) > 0 for *X*= *X*_*ϕ*_(*T*).  Let *ψ*(*t*)= *f*′(*X*_*ϕ*_(*t*)) + *φg*′(*X*_*ϕ*_(*t*)), where *f*′ and *g*′ are, respectively, the Jacobians of $f=\left[\begin{array}{c} f_{1}\left(x,y,z\right)\\ f_{2}\left(x,y,z\right)\\ f_{3}\left(x,y,z\right) \end{array}\right]$ and $\left[\begin{array}{c} -\sigma xy/f\left(y\right)\\ \sigma xy/f\left(y\right)\\ 0 \end{array}\right]$.

Let *Q*(*t*, *t*0), for 0 ≤ *t*_0_ ≤ *t* ≤ *T*, be a matrix function for which *Q*(*t*_0_, *t*_0_)=*I*  *d* and (∂*Q*(*t*, *t*_0_)/∂*t*)=*ψ*(*t*)*Q*(*t*, *t*_0_). Then, *DX*_0;*ϕ*_*h*=∫_0_^*T*^*Q*(*T*, *s*)*g*(*s*)*h*(*s*)d*s*.

**Lemma 4 .**

For every (*x*_0_, *y*_0_, *z*_0_) ∈ Π and (*x*, *y*, *z*) ∈ Π, there exists *k*(*T*, *x*, *y*, *z*; *x*_0_, *y*_0_, *z*_0_)  >  0, where Π is characterized as in (68).

**Proof**

Since a continuous control work *ϕ* is considered, the inequality (35) could be supplemented by these differential equations:

(70) $$\begin{array}{c} \left\{\begin{array}{c} x^{\prime }\phi \left(t\right)=f_{1}\left(x\phi \left(s\right),y\phi \left(s\right),z\phi \left(s\right)\right)\;-\sigma \phi \frac{x\phi \left(s\right)+\alpha y\phi \left(s\right)}{f\left(y\phi \left(s\right)\right)}x\phi \left(s\right),\\ y^{\prime }\phi \left(t\right)=f_{2}\left(x\phi \left(s\right),y\phi \left(s\right),z\phi \left(s\right)\right)\;+\sigma \phi \frac{x\phi \left(s\right)+\alpha y\phi \left(s\right)}{f\left(y\phi \left(s\right)\right)}x\phi \left(s\right),\\ z^{\prime }\phi \left(t\right)=f_{3}\left(x\phi \left(s\right),y\phi \left(s\right),z\phi \left(s\right)\right). \end{array}\right. \end{array}$$

Firstly, the rank of *D*_*X*_0_;*ϕ*_ is shown to be 3. Let

*h*(*t*)=(*χ*[*T* − *ε*, *T*](*t*)*f*(*yϕ*(*t*))/[*χϕ*(*t*)+*αyϕ*(*t*)]), *t* ∈ [0, *T*], where *χ* is a characteristic function. Since

(71) $$\begin{array}{c} Q\left(T,s\right)=I\;d+\psi \left(T\right)\left(s-T\right)+\frac{1}{2}\psi^{2}\left(T\right){\left(s-T\right)}^{2}+o\left({\left(s-T\right)}^{2}\right), \end{array}$$

we obtain *D*_*X*_0;*φh*__=*εV* − 1/2*ε*^2^*ψ*(*T*)*v*+1/6*ε*^3^*ψ*2(*T*)*v*+*o*(*ε*^3^), where $\nu =\left[\begin{array}{c} -\sigma \\ \sigma \\ 0 \end{array}\right]$, and

(72) $$\begin{array}{c} \psi \left(T\right).v=\left[\begin{array}{c} \frac{\sigma \left[\left(-x+y+\alpha z\right)\beta f\left(y\right)+\mu f^{2}\left(y\right)\;+\;x\left(y+\alpha z\right)\beta f^{\prime }\left(y\right)\right]}{f^{2}\left(y\right)}\\ -\left(\nu +\delta +\mu \right)\sigma \\ \frac{\beta \sigma \left[\left(x-y-\alpha z\right)f\left(y\right)-\;x\left(y+\alpha z\right)f^{\prime }\left(y\right)\right]}{f^{2}\left(y\right)} \end{array}\right]. \end{array}$$

Thus, *v*, *ψ*(*T*)*v*, and*ψ*^2^(*T*)*v* are straightly autonomous and the subsidiary *D*_*X*_0_;*ϕ*_ has a rank of 3.

Next, for any *X*_0_ ∈ Ω  and X ∈ Ω, we demonstrate the existence of a control work *ϕ* and *T* > 0 for which *X*_*φ*_(0)=*X*_0_ and *X*_*φ*_(*T*)=*X*. Set *ω*_*ϕ*_=*x*_*ϕ*_+*y*_*ϕ*_+*z*_*ϕ*_. Model (37) becomes

(73) $$\begin{array}{c} \left\{\begin{array}{c} g_{1}\left(x,w,z\right)=\Lambda -\mu x-\frac{\beta \left[z+\alpha \left(w-x-z\right)\right]}{f\left(z\right)}x+\gamma \left(N-\omega \right)-\sigma \varphi \frac{\left(z+\alpha \left(\omega -z-z\right)\right)St}{f},\\ g_{2}\left(x,w,z\right)=\Lambda +\mu z-\mu z-vz-\delta z-\left(\gamma +\mu \right)w,\\ g_{3}\left(x,w,z\right)=\eta \left(w-x-z\right)-\left(\mu +v+\delta \right)z. \end{array}\right. \end{array}$$

Let Π_0_={(*x*, *w*, *z*) ∈ :0 < *x*, *z* < Λ/*μ*, Λ/Λ+*μ* < *w* < Λ/*μ*and *x*, *z*, <*w*}. For any (*x*_0_, *w*_0_, *z*_0_) ∈  Π_0_ *an*  *d* .(*x*_1_, *w*_1_, *z*_1_)  ∈  Π_0_, it can be claimed that there exists a control function *ϕ* and *T* > 0 for which

(*x*_*ϕ*_(0), *w*_*ϕ*_(0), *z*_*ϕ*_(0))=(*x*_0_, *w*_0_, *z*_0_)and(*x*_*ϕ*_(*T*), *w*_*ϕ*_ (*T*), *z*_*ϕ*_(*T*))=(*x*_1_, *w*_1_, *z*1_1_). We create the function *ϕ* in the next steps. First of all, we determine a positive constant *T* and a differentiable function *w*_*ϕ*_ : [0, *T*]⟶(Λ/*μ*+*γ*, Λ/*μ*)_,_ for which

(74) $$\begin{array}{c} w_{\phi }\left(0\right)=w_{0},\\ w_{\phi }^{\prime }\left(T\right)=w_{1},\\ w_{\phi }^{\prime }\left(0\right)=g_{2}\left(x_{0},w_{0},z_{0}\right)=w_{0}^{d},\\ w_{\phi }^{\prime }\left(T\right)=g_{2}\left(x_{1},w_{1},z_{1}\right)=w_{T}^{d}\text{ and }\Lambda -\left(\mu +\gamma \right)w_{\phi }\left(t\right)<w_{\phi }^{\prime }\left(t\right)<\Lambda -\mu w_{\phi }\left(t\right)\mathrm{for}\;t\in \left[0,T\right]. \end{array}$$

For achieving this, the domain of the function *w*_*ϕ*_ is divided into 3 segments [0, *ε*], [*ε*, *T*_*ε*_] , and[*T* − *ε*, *T*], where 0 < *ε* < *T*/2. Let

(75) $$\begin{array}{c} \eta =\frac{1}{2}\min\left\{\omega_{0}-\frac{\Lambda }{\mu +\gamma },\omega_{1}-\frac{\Lambda }{\mu +\gamma },\frac{\Lambda }{\mu }-\omega_{0},\frac{\Lambda }{\mu }-\omega_{1}\right\}. \end{array}$$

If *ω*_*ϕ*_ ∈ (Λ/(*μ*+ *γ*)+*m*, Λ/*μ* − *m*), then we have the following equation:

(76) $$\begin{array}{c} \Lambda -\left(\mu +\gamma \right)\omega_{\phi }\left(t\right)<-\left(\mu +\gamma \right)m<0\text{ and }\Lambda -\mu \omega_{\phi }\left(t\right)>\mu m>0\text{ for }t\in \left[0,t\right]. \end{array}$$

Based on (41), a *C*^2^ function *ω*_*ϕ*_ : [0, *ε*]⟶(Λ/(*μ*+*γ*)+*m*, Λ/*μ* − *m*) can be obtained for which

(77) $$\begin{array}{c} \omega_{\phi }\left(0\right)=\omega_{0},\\ \omega_{\phi }^{\prime }\left(0\right)=\omega_{0}^{d},\\ \omega_{\phi }^{\prime }\left(\varepsilon \right)=0, \end{array}$$

where *ω*_*ϕ*_ satisfies (40) for *t* ∈ [0, *t*]. Similarly, a *C*^2^ function *ω*_*ϕ*_ : [*T* − *ε*, *T*]⟶(Λ/(*μ*+*γ*)+*m*, Λ/*μ* − *m*) is constructed so that

(78) $$\begin{array}{c} \omega_{\phi }\left(T\right)=\;\omega_{0},\omega_{\phi }^{\prime }\left(T\right)=\;\omega_{T}^{d},\omega_{\phi }^{\prime }\left(T-\varepsilon \right)=0, \end{array}$$

where *ω*_*ϕ*_ satisfies (40) for *t* ∈ [*T* − *ε*, *T*]. If we take *T* adequately big, we can spread the function *ω*_*ϕ*_ : [0, *ε*]∩[*T* − *ε*, *T*]⟶(Λ/(*μ*+*γ*)+*m*, Λ/*μ* − *m*) to a *C*^2^ function *ω*_*ϕ*_ on the whole segment [0, *T*] for which Λ − (*μ*+*γ*)*·ω*_*ϕ*_(*t*) < −(*μ*+*γ*)*m* < *ω*_*ϕ*_′(*t*) < *μm* < Λ − *μω*_*ϕ*_(*t*) for [*ε*, *T* − *ε*]. So, the function *ω*_*ϕ*_ satisfies (41) on [0, *T*].

As a result, a continuous function *φ* can be determined from the first equation of (38), while two functions *x*_*ϕ*_ and *z*_*ϕ*_ can be found where these functions satisfy the other equations in (38). This finishes the proof.

**Lemma 5 .**

Assume that *R*_0_^*s*^ > 1. For any density *g*, we get $\underset{t⟶\infty }{\lim}{∭}_{\Pi }P\left(t\right)g\left(x,y,z\right)dx\;dy\;dz=1$.

where Π is obtained from (13).

**Proof**

Following the proof of Lemma 5.6, we substitute *Z*_*t*_=*S*_*t*_+*E*_*t*_+*I*_*t*_. Then, model (3) can be rewritten as follows:

(79) $$\begin{array}{c} \left\{\begin{array}{c} dS_{t}=g_{1}\left(S_{t},Z_{t},I_{t}\right)dt-\frac{\sigma \left[It+\alpha \left(Z_{t}-S_{t}-I_{t}\;\right)\right]S_{t}}{f\left(I_{t}\right)}dBt,\\ dE_{t}=g_{2}\left(S_{t},Z_{t},I_{t}\right)dt-\frac{\sigma \left[It+\alpha \left(Z_{t}-S_{t}-I_{t}\;\right)S_{t}\right]}{f\left(I_{t}\right)}dBt,\\ dI_{t}=g_{3}\left(S_{t},Z_{t},I_{t}\right)dt, \end{array}\right. \end{array}$$

where *g*_1_(*x*, *w*, *z*),  *g*_2_(*x*, *w*, *z*), and *g*_3_(*x*, *w*, *z*) are introduced in (38). Since (*S*_*t*_, *E*_*t*_, *I*_*t*_) is a positive solution of model (5) with a probability of 1, and given *g*_2_, we have the following equation:

(80) $$\begin{array}{c} \Lambda -\left(\mu +\gamma \right)Z_{t}<\frac{dZ_{t}}{dt}<\Lambda -\mu Z_{t},t\in \left(0,\infty \right)\text{a}.s. \end{array}$$

Now, for almost every *w* ∈ Ω, we can show that there exists *t*_0_=*t*_0_(*w*) for which

(81) $$\begin{array}{c} \frac{\Lambda }{\mu +\gamma }<Z_{t}\left(w\right)<\frac{dZ_{t}}{dt}<\Lambda -\mu Z_{t}\;,\;for\;t>t_{0}. \end{array}$$

Actually, three cases exist.

(a) *Z*_0_ ∈ (Λ/*μ*+*γ*, Λ/*μ*): the conclusion is obvious from (45).
(b) *Z*_0_ ∈ (0, Λ/*μ*+*γ*): assume on the contrary that our claim is not true. Then, there would be Ω′ ∈ Ω with Prob (Ω′) > 0 for which *Z*_0_ ∈ (0, Λ/*μ*+*γ*). From (44), *Z*_*t*_(*w*) is carefully expanding on [0,∞) for any *w* ∈ Ω′ . Consequently,
  (82) $$\begin{array}{c} \underset{t⟶\infty }{\lim}Z_{t}\left(w\right)=\frac{\Lambda }{\mu +\gamma },\;w\in \Omega^{\prime }. \end{array}$$
From (43), we get $\underset{t⟶\infty }{\lim}S_{t}\left(w\right)=\underset{t⟶\infty }{\lim}I_{t}\left(w\right)=0,w\in \Omega^{\prime }$ and consequently $\underset{t⟶\infty }{\lim}E_{t}\left(w\right)=\Lambda /\mu +\gamma ,w\in \Omega^{\prime }.$ Thus, we get using the Itô formula,
  (83) $$\begin{array}{c} d\;\ln E_{t}=\left[\frac{\beta \alpha }{f\left(I_{t}\right)}S_{t}-\left(\mu +\eta \right)-\frac{\sigma^{2}\alpha^{2}S_{t}^{2}}{2f^{2}\left(I_{t}\right)}\right]\text{d}t+\frac{\sigma \alpha S_{t}}{f\left(I_{t}\right)}\text{d}B_{t}. \end{array}$$
Hence,
  (84) $$\begin{array}{c} \frac{\ln\;E_{t}-\ln\;E_{0}}{t}=\frac{1}{t}\int_{0}^{t}\left[\left[\frac{\beta \alpha }{f\left(I_{s}\right)}S_{s}-\left(\mu +\eta \right)-\frac{\sigma^{2}\alpha^{2}S_{s}^{2}}{2f^{2}\left(I_{s}\right)}\right]\right]+\frac{1}{t}\int_{0}^{t}\frac{\sigma \alpha S_{s}}{f\left(I_{s}\right)}\text{d}B_{s}. \end{array}$$
Since 1/*t*∫_0_^*t*^*σ*^2^*α*^2^*S*_*s*_^2^/*f*^2^(*I*_*s*_)d*s* ≤ *σ*^2^*α*^2^Λ^2^/*μ*^2^*f*^2^(0) < +*∞*, and using the strong law of large numbers for martingales [20], we get the following:
  (85) $$\begin{array}{c} \underset{t⟶\infty }{\lim}\frac{1}{t}\int_{0}^{t}\frac{\sigma \alpha S_{s}}{f\left(I_{s}\right)}\text{d}B_{s}=0. \end{array}$$
Therefore, taking into consideration the continuity of the functions *S*_*t*_, *E*_*t*_, *I*_*t*_, and *f*(*I*_*t*_), we obtain the following:
  (86) $$\begin{array}{c} \underset{t⟶\infty }{\lim}\frac{1}{t}\int_{0}^{t}\frac{\beta \alpha S_{s}}{f\left(I_{s}\right)}-\left(\mu +\eta \right)-\frac{\sigma^{2}\alpha^{2}S_{s}^{2}}{2f^{2}\left(I_{s}\right)}\text{d}s+\frac{1}{t}\int_{0}^{t}\frac{\sigma \alpha S_{s}}{f\left(I_{s}\right)}\text{d}B_{s}=-\left(\mu +\eta \right). \end{array}$$
This contradicts the limit $\underset{t⟶\infty }{\lim}\ln\;E_{t}-\ln\;E_{0}/t=0$, and thus, the claim is proved.
(c) *Z*_0_ ∈ (Λ/*μ*+*γ*, +*∞*): we use again a proof by contradiction with arguments similar to those in (b) to deduce that there is Ω′ ∈ Ω with Prob (Ω′) > 0 for which
  (87) $$\begin{array}{c} \underset{t⟶\infty }{\lim}Z_{t}\left(w\right)=\frac{\Lambda }{\mu },w\in \Omega^{\prime }. \end{array}$$

Using (44) and for any *w* ∈ Ω′, we get the following:

(88) $$\begin{array}{c} g_{2}\left(x,y,z\right)=\Lambda -\left(\mu +\delta +\nu \right)Z_{t}+\delta \left(E_{t}+S_{t}\right)+\gamma R_{t}+\nu S_{t}+\nu E_{t},\\ Z_{t}\left(w\right)=e^{-t\left(\mu +\delta +\nu \right)}\left(Z_{0}+\int_{0}^{t}e^{s\left(\mu +\delta +\nu \right)}\left(\Lambda +\delta \left(E_{t}+S_{t}\right)+\gamma R+\nu S_{t}+\nu E_{t}\right)\right)ds.\\ I_{t}\left(w\right)=e^{-t\left(\mu +\delta +\nu \right)}\left(R_{0}+\eta \int_{0}^{t}e^{s\left(\mu +\delta +\nu \right)}\left(Z_{s}\left(w\right)-S_{s}\left(w\right)-I_{t}\left(w\right)\right)\text{d}s\right). \end{array}$$

Hence, $\underset{t⟶\infty }{\lim}E_{t}\left(w\right)=0$, $\underset{t⟶\infty }{\lim}S_{t}\left(w\right)=0$, and $\underset{t⟶\infty }{\lim}I_{t}\left(w\right)=0$ for any *w* ∈ Ω′. Hence,

(89) $$\begin{array}{c} \underset{t⟶\infty }{\lim}\frac{\ln\;E_{t}-\ln\;E_{0}}{t}\\ =\underset{t⟶\infty }{\lim}\frac{1}{t}\int_{0}^{t}\left[\frac{\beta \alpha S_{s}}{f\left(I_{s}\right)}-\left(\mu +\eta \right)-\frac{\sigma^{2}\alpha^{2}S_{s}^{2}}{2f^{2}\left(I_{s}\right)}\text{d}s\right]+\frac{1}{t}\int_{0}^{t}\frac{\sigma \alpha S_{s}}{f\left(I_{s}\right)}\text{d}B_{s}\\ =\frac{\beta \alpha \Lambda }{\mu f\left(I_{0}\right)}-\left(\mu +\eta \right)-\frac{\sigma^{2}\alpha^{2}\Lambda^{2}}{2\mu^{2}f^{2}\left(0\right)}\\ =\left(\mu +\eta \right)\left[\frac{2\mu f\left(0\right)\beta \alpha \Lambda }{2\mu^{2}f^{2}\left(0\right)\left(\mu +\eta \right)}-1\right]>0,a.s.\text{on }\Omega^{\prime }. \end{array}$$

This is contradictory to the assumption that lim_*t*⟶*∞*_*I*_*t*_=0 a.s. and the claim follows. Remark 7: from Lemmas 4 and 5, we realize that when the Fokker–Planck equation (11) has a stationary solution *U*_*∗*_, then sup *U*_*∗*_ = Π.

**Lemma 6 .**

Assume that *R*_0_^*s*^ > 1, the semigroup {*P* (*t*)} *t* ≥ 0 is either sweeping with respect to minimal sets or asymptotically stable.

**Proof**

By Lemma 3, the operator family {*P* (*t*)} *t* ≥ 0 is a fundamental Markov semigroup with a constant kernel *k*(*t*, *x*, *y*, *z*, *x*0, *y*0, *z*0) for *t* > 0. Then, the appropriation of (*S*_*t*_, *E*_*t*_, *I*_*t*_) possesses a density *U*(*x*, *y*, *z*, *t*), which fulfills (19). From Lemma 5, the semigroup {P (*t*)} *t* ≥ 0 can be restricted to the space *L*0 (Π). As indicated by Lemma 4, for each *f* ∈ D, we have the following:

(90) $$\begin{array}{c} \int_{0}^{\infty }P_{t}f\text{d}t>0,a.s. \end{array}$$

Thus, from Lemma 1, the semigroup {*P*(*t*)}, *t* ≥ 0 is asymptotically stable or is sweeping with respect to minimal sets.

## 5. Numerical Simulation Results

We demonstrate here the results of simulations of the deterministic and the stochastic models. These simulations clarify the effects of stochasticity on the epidemic dynamics. The simulations of the stochastic model are performed following the Milstein strategy [45]. We simulate the SDE solutions with *f*(*I*)=1+*aI*^2^. For the convenience of display, the simulation is set as 100 times 100 in the space-time range, the abscissa represents the time, and the ordinate represents the number of patients. The simulations can help us to investigate how the ecological perturbations and the harmfully idle periods influence the spread of epidemics. In particular, we consider the global characteristics of a general SDE model with infection forces for both the deterministic case (without infection forces) and the stochastic case (with infection forces). In the first set of simulations, the parameters of the stochastic model are set as follows: *λ* = 0.23, *μ* = 0.01, *α* = 0.36, *β* = 0.52, *γ* = 0.45, *σ* = 0.6, *δ* = 0.31, *v* = 0.13, *η* = 0.25, and *a* = 0.1 (see Figure 1).

The results in Figure 1 are based on a stochastic reproduction number of *R*_0_^*s*^ = 2.8917, which is more than 1. We take the initial conditions to be (*S*_*t*_, *E*_*t*_, *I*_*t*_, *R*_*t*_) = (0.9, 0.06, 0.04, 0). It is easy to see that the system is oscillating. Next, we study how environmental oscillations affect the spread of epidemics by reviewing the global dynamics of the general SEIRS model.

We take the parameter values as follows: *λ* = 0.001, *µ* = 0.01, *α* = 0.35, *β* = 0.6, *γ* = 0.05, *σ* = 0.15, *a* = 5, *δ* = 0.05, *ν* = 0.6, *η* = 0.33, *R*_0_^*s*^ = 1.5329 > 1, and *R*_0_ = 0.9877 < 1. The simulation results for the deterministic model are shown in Figure 2. It is easy to see that the deterministic system is stable. To understand the influence of the environmental noise on the system, we increase gradually the disturbance parameter *σ* = 0.15, 0.35, 0.55, and 0.75, while keeping the other parameters unchanged.

The results are shown in Figures 3–6. From these figures, we can conclude that increasing the intensity of the system disturbance gradually leads naturally to more disturbances of the relevant quantities. However, when the noise level is above a certain threshold, these quantities are severely disturbed at the beginning but then stabilize gradually.

Figures 7–9 discuss the influence of the change in a variable on the system. The conclusion is that with the increase in *α*, the system has stronger disturbance and worse control ability. Therefore, the incubation period is an important variable in disease control. The existence of the incubation period will lead to the difficulty of disease control.

We computed the time series and confidence intervals of each variable, as shown in Figures 10 and 11. From the simulations, we can see that the stability of the system is affected, and the fluctuation range is big. For this set of simulations, we set the parameters as follows: *λ* = 0.001, *μ* = 0.01, *α* = 0.75, *β* = 0.1, *γ* = 0.25, *σ* = 0.35, *a* = 0.001, *δ* = 0.05, *ν* = 0.1, and *η* = 0.33.

There are many variables in the system. We only discussed several representative variables in detail. In the actual disease control, we can discuss the influence of each variable on the system, so as to better control the spread of disease.

Several groups of simulation results show that the conclusion of this study is correct. In the actual disease model control, we should pay attention to the types of diseases and fully consider the interference of random factors. The establishment of control variables in this study can provide basic theoretical basis and model reference for the simulation of subsequent infectious disease models.

## 6. Conclusions

Worldwide populations have been largely and negatively impacted by infectious disease outbreaks, which had detrimental effects socially and economically [5]. Individual responses go from maintaining a safe distance from infected people to wearing defensive covers, or taking immunizations. Intervention approaches seek to change human behavior, to decrease the contact rates of susceptible people [6]. Compared with other models, such as literature [21, 46], this model establishes a four-variable random infectious disease model, which adds the influence of incubation period, which is more in line with reality. At present, there are few studies on relevant theories and simulation.

Natural infection forces affect the spread of epidemics. In this study, we investigated the components of a stochastic SEIRS model with a general contamination force. The stochastic effects were considered by incorporating a multiplicative background noise in the development conditions of both the susceptible and exposed populations.

Our investigations uncover two important perspectives. Firstly, the generation number *R*_*o*_^*s*^ can be used to control the stochastic elements of a SDE model based on the Markov semigroup assumptions. If *R*_*o*_^*s*^ < 1, and with gentle additional conditions, the SDE framework has a disease-free solution set, which implies the eradication of the epidemic with a likelihood of 1. When *R*_*o*_^*s*^ > 1, and again under mild additional conditions, the SDE framework has an endemic equilibrium. This prompts the stochastic persistence of the disease.

The number *R*_0_^*S*^ is the main control variable of random infectious disease model control, which should be considered in practice. In addition, the change in initial value may also lead to uncontrollable results of the system, which brings greater challenges to infectious disease control.

## Figures and Tables

**Figure 1:** Temporal functions of *S*(*t*), *E*(*t*), *I*(*t*), and *R*(*t*) for the stochastic model.

**Figure 2:** Temporal functions of *S*(*t*), *E*(*t*), *I*(*t*), and *R*(*t*) for the deterministic model with initial values of (*S*_0_, *E*_0_, *I*_0_, *R*_0_) = (0.9, 0.06, 0.04, 0).

**Figure 3:** Temporal functions of *S*(*t*), *E*(*t*), *I*(*t*), and *R*(*t*) for the stochastic model with initial values (*S*_0_, *E*_0_, *I*_0_, *R*_0_) = (0.9, 0.06, 0.04, 0), *σ* = 0.15, and *R*_0_^*s*^ = 1.4286 > 1.

**Figure 4:** Temporal functions of *S*(*t*), *E*(*t*), *I*(*t*), and *R*(*t*) for the stochastic model with initial values (*S*_0_, *E*_0_, *I*_0_, *R*_0_) = (0.9, 0.06, 0.04, 0), *σ* = 0.35, and *R*_0_^*s*^ = 1.4062 > 1.

**Figure 5:** Temporal functions of *S*(*t*), *E*(*t*), *I*(*t*), and *R*(*t*) for the stochastic model with initial values (*S*_0_, *E*_0_, *I*_0_, *R*_0_) = (0.9, 0.06, 0.04, 0), *σ* = 0.55, and *R*_0_^*s*^ = 1.2035 > 1.

**Figure 6:** Temporal functions of *S*(*t*), *E*(*t*), *I*(*t*), and *R*(*t*) for the stochastic model with initial values (*S*_0_, *E*_0_, *I*_0_, *R*_0_) = (0.9, 0.06, 0.04, 0), *σ* = 0.75, and *R*_0_^*s*^ = 0.9108 < 1.

**Figure 7:** Temporal functions of *S*(*t*), *E*(*t*), *I*(*t*), and *R*(*t*) for the stochastic model with initial values (*S*_0_, *E*_0_, *I*_0_, *R*_0_) = (0.9, 0.06, 0.04, 0), *α* = 0.55, and *R*_0_^*s*^ = 6.7825.

**Figure 8:** Temporal functions of *S*(*t*), *E*(*t*), *I*(*t*), and *R*(*t*) for the stochastic model with initial values (*S*_0_, *E*_0_, *I*_0_, *R*_0_) = (0.9, 0.06, 0.04, 0), *α* = 0.8, and *R*_0_^*s*^ = 1.4329.

**Figure 9:** Temporal functions of *S*(*t*), *E*(*t*), *I*(*t*), and *R*(*t*) for the stochastic model with initial values (*S*_0_, *E*_0_, *I*_0_, *R*_0_) = (0.9, 0.06, 0.04, 0), *α* = 1.02, and *R*_0_^*s*^ = 67.5118.

**Figure 10:** Temporal functions of *S*(*t*), *E*(*t*), *I*(*t*), and *R*(*t*) for the stochastic model with initial values (*S*_0_, *E*_0_, *I*_0_, *R*_0_) = (0.9, 0.06, 0.04, 0).

**Figure 11:** Temporal functions of *S*(*t*), *E*(*t*), *I*(*t*), and *R*(*t*) for the stochastic model with initial values (*S*_0_, *E*_0_, *I*_0_, *R*_0_) = (0.9, 0.06, 0.04, 0) and confidence intervals.

## Data Availability

The data used to support the findings of this study are included within the article.

## References

[1] Buseh A. G., Stevens P. E., Bromberg M., Kelber S. T. (2015). The Ebola epidemic in West Africa: challenges, opportunities, and policy priority areas. *Nursing Outlook*.

[2] Li H., Ying T., Yu F., Lu L., Jiang S. (2015). Development of therapeutics for treatment of Ebola virus infection. *Microbes and Infection*.

[3] Ye L., Yang C. (2015). Development of vaccines for prevention of Ebola virus infection. *Microbes and Infection*.

[4] Fenner E., Henderson D. A. (2008). Summary of probable SARS cases with on set of illness from1 November 2002 to31July 2003. https://www.who.int/publications/m/item/summary-of-probable-sars-cases-with-onset-of-illness-from-1-november-2002-to-31-july-2003.

[5] Báez-Santos Y. M., Sarah E., John S., Mesecar A. D. (2015). The SARS coronavirus papainlike protease: structure, function and inhibition by designed antiviral compounds. *Antiviral Research*.

[6] Mahajan M., Bhattacharjya S. (2015). NMR structures and localization of the potential fusion peptides and the pre-transmembrane region of SARS-CoV: i. *Biochimica et Biophysica Acta (BBA) - Biomembranes*.

[7] Shimamoto Y., Hattori Y., Kobayashi K. (2015). Fused-ring structure of decahydroisoquinolin as a novel scaffold for SARS 3CL protease inhibitors. *Bioorganic & Medicinal Chemistry*.

[8] Mao H., Guo B., Wang F. (2015). A study of family clustering in two young girls with novel avian influenza A (H7N9) in Dongyang, Zhejiang Province, in 2014. *Journal of Clinical Virology*.

[9] Zhu W., Shu Y. (2015). Genetic tuning of avian influenza A (H7N9) virus promotes viral fitness within different species. *Microbes and Infection*.

[10] Spackman E., Pantin-Jackwood M., Swayne D. E., Suarez D. L., Kapczynski D. R. (2015). Impact of route of exposure and challenge dose on the pathogenesis of H7N9 low pathogenicity avian influenza virus in chickens. *Virology*.

[11] Hu W., Zhang W., Huang X., Clements A., Mengersen K., Tong S. (2015). Weather variability and influenza A (H7N9) transmission in Shanghai, China: a Bayesian spatial analysis. *Environmental Research*.

[12] Wu H., Lu R., Peng X. (2015). Novel reassortant highly pathogenic H5N6 avian influenza viruses in poultry in China. *Infection, Genetics and Evolution*.

[13] Li Q., Wang X., Gao Z. (2015). Novel reassortant H5N5viruses bind to a human-type recept or as afact or in pan-demic risk. *Veterinary Microbiology*.

[14] Gray A., Greenhalgh D., Hu L., Mao X., Pan J. (2011). A stochastic differential equation SIS epidemic model. *SIAM Journal on Applied Mathematics*.

[15] Tornatore E., Maria Buccellato S., Vetro P. (2005). Stability of a stochastic SIR system. *Physica A: Statistical Mechanics and Its Applications*.

[16] Tornatore E., Vetro P., Buccellato S. M. (2014). SIVR epidemic model with stochastic perturbation. *Neural Computing & Applications*.

[17] Ji C., Jiang D. (2014). Threshold behaviour of a stochastic SIR model. *Applied Mathematical Modelling*.

[18] Lahrouz A., Omari L. (2013). Extinction and stationary distribution of a stochastic SIRS epidemic model with non-linear incidence. *Statistics & Probability Letters*.

[19] Zhao Y., Jiang D., O’Regan D. (2013). The extinction and persistence of the stochastic SIS epidemic model with vaccination. *Physica A: Statistical Mechanics and Its Applications*.

[20] Lin Y., Jiang D., Wang S. (2014). Stationary distribution of a stochastic SIS epidemic model with vaccination. *Physica A: Statistical Mechanics and Its Applications*.

[21] Cai Y., Kang Y., Banerjee M., Wang W. (2015). A stochastic SIRS epidemic model with infectious force under intervention strategies. *Journal of Differential Equations*.

[22] Mummert A., Otunuga O. M. (2019). Parameter identification for a stochastic SEIRS epidemic model: case study influenza. *Journal of Mathematical Biology*.

[23] Norden R. H. (1992). On the distribution of the time to extinction in the stochas-tic logistic population model. *Advances in Applied Probability*.

[24] Gumel A. B., Ruan S., Day T. (2004). Modelling strategies for controlling SARS outbreaks. *Proceedings of the Royal Society of London-Series B: Biological Sciences*.

[25] Dalal N., Greenhalgh D., Mao X. (2008). A stochastic model for internal HIV dynamics. *Journal of Mathematical Analysis and Applications*.

[26] Dalal N., Greenhalgh D., Mao X. (2007). A stochastic model of AIDS and condom use. *Journal of Mathematical Analysis and Applications*.

[27] Talkibing H. Y., Diakarya B., Fabrice O. (2019). Stochastic approach in epidemic modeling using the SEIRS. *European Journal of Pure and Applied Mathematics*.

[28] Xiao D., Ruan S. (2007). Global analysis of an epidemic model with nonmonotone incidence rate. *Mathematical Biosciences*.

[29] Wang W. (2006). Epidemic models with nonlinear infection forces. *Mathematical Biosciences and Engineering*.

[30] Ruan S., Wang W. (2003). Dynamical behavior of an epidemic model with a nonlinear incidence rate. *Journal of Differential Equations*.

[31] van den Driessche P., Watmough J. (2002). Reproduction numbers and sub-threshold endemic equilibria for compartmental models of disease transmission. *Mathematical Biosciences*.

[32] Komorowski T., Tyrcha J. (1989). Asymptotic properties of some Markov operators. *Bulletin of the Polish Academy of Sciences-Mathematics*.

[33] Lasota A., Mackey M. C. (1994). *Chaos, Fractals, and Noise: Stochastic Aspects of Dynamics*.

[34] Rudnicki R. (1995). On asymptotic stability and sweeping for Markov operators. *Bulletin of the Polish Academy of Sciences-Mathematics*.

[35] Kadanoff L. P. (2000). *Statistical Physics: Statics, Dynamics, and Renormalization*.

[36] Rudnicki R. (2000). Markov operators: applications to diffusion processes and population dynamics. *Applicationes Mathematicae*.

[37] Rudnicki R., Pichór K., Tyran-Kamińska M. (2002). Markov semigroups and their applications. *Dynamics of Dissipation*.

[38] Rudnicki R. (2003). Long-time behaviour of a stochastic prey-predator model. *Stochastic Processes and Their Applications*.

[39] LaSalle J. P. (1987). The stability of dynamical systems. *Society for Industrial and Applied Mathematics*.

[40] Lyapunov A. M. (1992). The general problem of the stability of motion. *International Journal of Control*.

[41] Arous G. B., Léandre R. (1991). Décroissance exponentielle du noyau de la chaleur sur la diagonale (II). *Probability Theory and Related Fields*.

[42] Mao X. (1997). *Stochastic Differential Equations and Their Applications*.

[43] Bell D. R. (2006). *The Malliavin Calculus*.

[44] Stroock D. W., Varadhan S. R. S. On the support of diffusion processes with applications to the strong maximum principle.

[45] Murray J. D., Stanley E. A., Brown D. L. (1986). On the spatial spread of rabies among foxes. *Proceedings of the Royal Society of London-Series B: Biological Sciences*.

[46] Busenberg S., van den P. (2013). Driessvhe properties of swiching diffusion epidemic model with varying population size. *Applied Mathematics and Computation*.

